The article "Physio-metabolic and clinical consequences of wearing face masks—Systematic review with meta-analysis and comprehensive evaluation" was retracted in 2023. Reasons: concerns about the data; concerns about the results or conclusions.

# Physio-metabolic and clinical consequences of wearing face masks—Systematic review with meta-analysis and comprehensive evaluation

**DOI:** 10.3389/fpubh.2023.1125150

**Published:** 2023-04-05

**Authors:** Kai Kisielinski, Oliver Hirsch, Susanne Wagner, Barbara Wojtasik, Stefan Funken, Bernd Klosterhalfen, Soumen Kanti Manna, Andreas Prescher, Pritam Sukul, Andreas Sönnichsen

**Affiliations:** ^1^Orthopaedic and Trauma Surgery, Clinical Medicine, Private Practice, Düsseldorf, Germany; ^2^Department of Psychology, Fachhochschule für Oekonomie und Management (FOM) University of Applied Sciences, Siegen, Germany; ^3^Veterinary Medicine, Wagner Medical Science Liason (MSL) Management, Blankenfelde-Mahlow, Germany; ^4^Department of Genetics and Biosystematics, Faculty of Biology, University of Gdańsk, Gdansk, Poland; ^5^Internal Medicine, Clinical Medicine, Private Practice, Moers, Germany; ^6^Institute of Pathology, Dueren Hospital, Dueren, Germany; ^7^Biophysics and Structural Genomics Division, Saha Institute of Nuclear Physics, Kolkata, India; ^8^Institute of Molecular and Cellular Anatomy (MOCA), Rhine-Westphalia Technical University of Aachen, Aachen, Germany; ^9^Rostock Medical Breath Research Analytics and Technologies (ROMBAT), Department of Anesthesiology and Intensive Care, University Medicine Rostock, Rostock, Germany; ^10^Internal Medicine, Clinical Medicine, Private Practice, Gesundheit für Österreich e.V. (Health for Austria), Vienna, Austria

**Keywords:** masks and N95 respirators, surgical mask, adverse (side) effects, long-term adverse effects, health risk assessment, MIES syndrome, risk-benefit, mask

## Abstract

**Background:**

As face masks became mandatory in most countries during the COVID-19 pandemic, adverse effects require substantiated investigation.

**Methods:**

A systematic review of 2,168 studies on adverse medical mask effects yielded 54 publications for synthesis and 37 studies for meta-analysis (on *n* = 8,641, *m* = 2,482, *f* = 6,159, age = 34.8 ± 12.5). The median trial duration was only 18 min (IQR = 50) for our comprehensive evaluation of mask induced physio-metabolic and clinical outcomes.

**Results:**

We found significant effects in both medical surgical and N95 masks, with a greater impact of the second. These effects included decreased SpO_2_ (overall Standard Mean Difference, SMD = −0.24, 95% CI = −0.38 to −0.11, *p* < 0.001) and minute ventilation (SMD = −0.72, 95% CI = −0.99 to −0.46, *p* < 0.001), simultaneous increased in blood-CO_2_ (SMD = +0.64, 95% CI = 0.31–0.96, *p* < 0.001), heart rate (N95: SMD = +0.22, 95% CI = 0.03–0.41, *p* = 0.02), systolic blood pressure (surgical: SMD = +0.21, 95% CI = 0.03–0.39, *p* = 0.02), skin temperature (overall SMD = +0.80 95% CI = 0.23–1.38, *p* = 0.006) and humidity (SMD +2.24, 95% CI = 1.32–3.17, *p* < 0.001). Effects on exertion (overall SMD = +0.9, surgical = +0.63, N95 = +1.19), discomfort (SMD = +1.16), dyspnoea (SMD = +1.46), heat (SMD = +0.70), and humidity (SMD = +0.9) were significant in *n* = 373 with a robust relationship to mask wearing (*p* < 0.006 to *p* < 0.001). Pooled symptom prevalence (*n* = 8,128) was significant for: headache (62%, *p* < 0.001), acne (38%, *p* < 0.001), skin irritation (36%, *p* < 0.001), dyspnoea (33%, *p* < 0.001), heat (26%, *p* < 0.001), itching (26%, *p* < 0.001), voice disorder (23%, *p* < 0.03), and dizziness (5%, *p* = 0.01).

The article "Physio-metabolic and clinical consequences of wearing face masks—Systematic review with meta-analysis and comprehensive evaluation" was retracted in 2023. Reasons: concerns about the data; concerns about the results or conclusions.

**Discussion:**

Masks interfered with O_2_-uptake and CO_2_-release and compromised respiratory compensation. Though evaluated wearing durations are shorter than daily/prolonged use, outcomes independently validate mask-induced exhaustion-syndrome (MIES) and down-stream physio-metabolic disfunctions. MIES can have long-term clinical consequences, especially for vulnerable groups. So far, several mask related symptoms may have been misinterpreted as long COVID-19 symptoms. In any case, the possible MIES contrasts with the WHO definition of health.

**Conclusion:**

Face mask side-effects must be assessed (risk-benefit) against the available evidence of their effectiveness against viral transmissions. In the absence of strong empirical evidence of effectiveness, mask wearing should not be mandated let alone enforced by law.

**Systematic review registration:**

https://www.crd.york.ac.uk/prospero/display_record.php?ID=CRD42021256694, identifier: PROSPERO 2021 CRD42021256694.

## Introduction

In most countries, the uses of medical face masks have been restricted to professionals for decades (1). In the health-care setting, masks constituted a mandatory self-protective and third-party protective measure for medical personnel prior to COVID-19 pandemic (2) based on the assumption of efficacy of masks in reducing transmission of pathogens, especially bacteria (3). The effectiveness of masks in all healthcare settings was debatable even before 2020 (4, 5). In 2020, many scientists and leaders started to believe that the use of masks could also provide protection against viral transmission, although evidence for the effectiveness of this measure was only weak (6). Since the pandemic began, a large number of studies tried to assess the antiviral effectiveness of masks, with hardly conclusive results (7, 8).

During the 2019 SARS-CoV-2 outbreak face masks were deployed as a mandatory public health measure for the general population in many countries around the world (9), making them one of the most important universal life-style attributes that directly affect how we breathe. As with any other preventive measure and/or intervention, masks also have specific disadvantages. While certain properties may have justified their invention and application in the past, e.g., retention of bacteria during surgical wound care and operations (1, 2), at present the question needs to be addressed as to the long-term effects widespread mask wearing may have on normal breathing. It is noteworthy that the compulsory wearing of masks for the entire population provided good research conditions for studying the adverse effects of mask wearing (10–17). Various volatile metabolites are produced through biochemical and metabolic pathways and their concentrations in exhaled breath provide immediate physiological (18, 19), metabolic (20, 21), and pathological (22, 23) signs with the possibility of monitoring various processes and interventions including therapies (24, 25). A recent observational study reported continuous respiratory and hemodynamic changes along with corresponding alteration in exhaled volatile metabolites (viz. potentially originate at the cellular/organ levels and *via* microbial metabolic processes) and has raised significant concerns upon the immediate, progressive, transient, and long-term side-effects of FFP2/N95 and surgical masks in adults (aged between 20 and 80 years) at rest (26). Recently, the harmful effects of masks were highlighted in a large scoping (non-systematic) review (14) that has summoned for a systematic review with comprehensive evaluation of mask induced adverse consequences.

The article "Physio-metabolic and clinical consequences of wearing face masks—Systematic review with meta-analysis and comprehensive evaluation" was retracted in 2023. Reasons: concerns about the data; concerns about the results or conclusions.

Though some important systematic reviews regarding masks and their effects already exist (27–30), they are predominantly restricted to healthy and sportive individuals (27, 29). Due to the exclusion of children, pregnant women and diseased patients from these evaluations and conclusions (28, 31), the reviews do not provide sufficient evidence that masks can be safely used the general population. Moreover, the application of fixed statistical models (27), use of narratives rather than quantitative analysis and statistics (despite claiming to be systematic) (32), focus on health care workers (31), as well as comparing the different mask types without any baseline/control group (31) were ubiquitous limitations of those studies. Physiological systematic reviews based purely on physiological effects of masks limit data interpretations to normal physio-metabolic fluctuations i.e., beyond the domain of pathophysiological compensatory mechanisms (especially in the older individuals and those with diminished compensatory reserves) and/or acute/chronic subliminal changes in the human microbiome (28, 30). In addition, other studies have not addressed subjective prevalence of symptoms and discomfort during mask use and concomitant physical changes such as heat and temperature in detail (27, 29). Therefore, the systematic reviews available to date neither address possible symptoms of mask use for the general population nor their exact prevalence. In addition, the transferability of the outcomes of said systematic reviews to the general population is very limited and they do not fulfill the actual requirements of clinical and inclusive evaluation, especially from the views and perspectives of medical practitioners.

The article "Physio-metabolic and clinical consequences of wearing face masks—Systematic review with meta-analysis and comprehensive evaluation" was retracted in 2023. Reasons: concerns about the data; concerns about the results or conclusions.

Including young, old, healthy and ill people to the systematic analysis of physiological, metabolic, and clinical data would increase our understanding about the impact of mask-wearing on the general population. In contrast to the above-indicated studies, our systematic review is aimed to quantify the biochemical/metabolic, physical, physiological changes along with the appearance of subjective and clinical symptoms in face mask users and analyze them from a clinician's and physician's holistic perspective.

## Materials and methods

### Registration

This meta-analysis was registered with the international prospective register of systematic reviews (PROSPERO) under the record CRD42021256694 at the National Institute for Health Research (NIHR) and performed in accordance with the Preferred Reporting Items for Systematic Reviews and Meta-Analyses (PRISMA) Statement (33).

### Inclusion and exclusion criteria

The aim was to study adverse effects of face masks on metabolic, physiological, physical, psychological, and individualized parameters. The use of cloth masks, surgical masks and N95/FFP-2 masks were the intervention of interest. Humans of all ages and genders, who were evaluated in controlled intervention studies and observational studies have been included in our comprehensive evaluation. Case reports, narrative reviews, case series and expert opinions were excluded. The main outcomes considered were peripheral oxygen saturation (SpO_2_), carbon dioxide levels in blood, temperature, humidity, heart rate, respiratory rate, tidal volume and minute ventilation, blood pressure, exertion, dyspnea, discomfort, headache, skin changes, itching, psychological stress, and symptoms during the use of face masks.

### Literature retrieval strategy

First, a comprehensive search term was developed. Then, PubMed, Embase, and Cochrane Library databases were searched. The search was performed until 31st December 2021. There were no restrictions in publication date. Literature that was neither English nor German language was excluded. Additionally, forward-looking data was considered for discussion, but not included in the meta-analysis. Preprints that have been published in journals in the meantime have been given the appropriate references.

The article "Physio-metabolic and clinical consequences of wearing face masks—Systematic review with meta-analysis and comprehensive evaluation" was retracted in 2023. Reasons: concerns about the data; concerns about the results or conclusions.

### Literature screening and data extraction

Search terms were created according to the criteria defined in the PICO scheme (34). The specific search terms were: (face mask^*^ [tw], FFP1 [tw] FFP2 [tw], FFP3 [tw], N99 [tw], N97 [tw], N95 [tw], respiratory protective device^*^ [tw], air-purifying respirator^*^ [tw], surgical mask^*^ [tw]) and (risk^*^ or adverse effect^*^ [tw], adverse event^*^ [tw], side effect^*^ [tw], psycho^*^ [tw], hypoxia [tw], hypercapnia [tw], headache [tw], dead space [tw], safety [tw], carbon dioxide [tw]), not infants, not neonatal, not newborn, not endoscopy, not CPAP, not intubate^*^, not propofol, not resuscitation, not mechanical ventilation [tw], not fetus. The asterisk in the search algorithm here “^*^” stands for the extension of the spelling with different possible letter combinations (e.g., face mask^*^ with ^*^= s, or ^*^=ed, or ^*^=ing). The abbreviation “[tw]” stands for title word.

The retrieved titles and abstracts were then screened and assessed for predefined inclusion criteria by at least three authors. Study design, methodology, interventions, primary and secondary outcomes and language were evaluated using the web-based program Rayyan—a web and mobile app for systematic reviews (35). Full texts of all potentially relevant articles were independently assessed for inclusion by two authors. Full-text exclusions and reasons have been documented. Data of included full texts were extracted: Author and year, type of study, aim of the study, intervention/control, sample size, follow-up, outcomes, funding, setting/country, age, sex, comorbidities, medications, functional status and cognitive status of participants, results, main findings, and limitations. Descriptive data was extracted by one author and checked by another author. If discrepancies occurred or authors disagreed, a senior author was involved in and a consensus was found (36).

### Risk of bias assessment of the included studies

The quality assessments were carried out using various tools, depending on the type of study. If systematic reviews and meta-analyses were included, these were assessed using the AMSTAR-2 checklist (37). Interventional studies were examined using the manual “Assessment of the risk of bias in clinical studies” from the Cochrane Collaboration (Cochrane RoB-2) (38). Observational studies were checked with the CASP (Critical Appraisal Skills Program) using standardized forms (39).

The article "Physio-metabolic and clinical consequences of wearing face masks—Systematic review with meta-analysis and comprehensive evaluation" was retracted in 2023. Reasons: concerns about the data; concerns about the results or conclusions.

### Statistical analysis

A meta-analysis was carried out, if at least two studies with the same research question were found among the randomized, non-randomized controlled trials, and observational studies. A subgroup analysis was conducted, where possible, for different mask types (N95/surgical) and even compared the mask types with each other (N95 vs. surgical mask). The program “RevMan-5.4.1,” which was developed for Cochrane Reviews was used. As we anticipated a considerable between-study heterogeneity -the random effects model was used to pool effect sizes (40). The results were graphically depicted in forest plots. Subgroup analyses were performed and a *Q*-test was calculated to examine significant subgroup differences. Study heterogeneity was assessed using Cochrane's *Q*-test, T2 according to DerSimonian and Laird (41), and *I*^2^ according to Higgins and Thompson (42). Where possible, a funnel plot was created to investigate publication bias. If this showed an abnormal result and there were at least 10 studies evaluating the same question, Egger's test (43) was carried out.

For the analysis of metabolic and physiological changes all controlled intervention studies in which measurements were taken during physical activity with face masks were included. We excluded resting conditions since these are not particularly representative for real life settings. Additionally, we excluded pre-post studies to ensure study-comparability. In addition, by excluding rest situations of the mostly healthy study participants, our approach was able to represent the possible effects better in older adults and ill individuals (e.g., with compromised compensation mechanisms), all of whom are a significant part of the general population. This also helped to reduce heterogeneity (*I*^2^). Neither for the results of the systolic blood pressure (SBP) nor the temperature did we follow this approach. Studies in which measurements were taken during rest and moderate physical activity were included in the meta-analysis of the physical outcome on SBP to obtain an evaluable number of studies and to ensure a better comparability and lower heterogeneity (exclusion of heavy load exercise conditions). In order to gather more available data for evaluating the temperature, we included two pre-post studies containing a resting condition using valid methodology and exact temperature measurements. This clearly reduced the heterogeneity index *I*^2^. For the meta-analysis of the resultant CO_2_-blood-content the joint evaluation of different experimental CO_2_ measurements (PtCO_2_, ETCO_2_, and PaCO_2_) in mmHg was justified by the following facts:

1) “ETCO_2_ and PtCO_2_ measurements both provide an estimation of PaCO_2_” (44).
2) “End-tidal CO_2_ (ETCO_2_) has been considered as a reliable estimate of arterial PCO_2_, in healthy subjects” (45).
3) “PtCO_2_ reliably reflects PaCO_2_, irrespective of sensor location” (46).
4) “Transcutaneous CO_2_ (PtCO_2_) devices provide another option for the continuous non-invasive estimation of PaCO_2_, overcoming the limitations posed by end-tidal CO_2_ analysis” (45).
5) “ETCO_2_ monitoring tends to underestimate PaCO_2_ levels” (44).

The article "Physio-metabolic and clinical consequences of wearing face masks—Systematic review with meta-analysis and comprehensive evaluation" was retracted in 2023. Reasons: concerns about the data; concerns about the results or conclusions.

For meta-analysis of measured sensations, all studies in which measurements were mainly taken during physical activity were included. This helped to ensure comparability, lower heterogeneity and the above mentioned aims to draw conclusions on the general population under conditions resembling real life settings. However, an exemption was made for the sensation “discomfort:” To allow evaluable study numbers, we included one pre-post study with resting condition, however, with valid methodology and exact discomfort evaluations (47). Even if this study had not been included, the result would be significant and unambiguous, however with a slightly larger 95% CI.

Our systematic review also referenced studies aiming to assess the prevalence of sensations and symptoms under mask use. Therefore, we conducted an additional meta-analysis of these observational studies to document the pooled prevalence in mask use. Prevalence was calculated as total number of symptoms per 100 mask wearers. In studies where the standard error (SE) was not reported, we calculated it from the prevalence using the following formula: SE = √p (1-p) / n with a 95% CI = p ± 1.96 X SE; where, p = Prevalence. This statistical approach to quantify a pooled prevalence from observational studies has been previously reported (48). Meta-analysis was performed using RevMan (Version 5.4.1). The heterogeneity of each meta-analysis was assessed and then the random effects model was used to calculate the pooled prevalence. We conducted subgroup analysis where possible for mask type (N95/surgical). Funnel plots were used to study the possibility of publication bias as described above.

The inclusion of observational studies, particularly for the prevalence analysis in our meta-analysis is justified because these are particularly suitable to investigate exposures that are difficult or impossible to investigate in randomized controlled trials (RCTs), e.g., air pollution or smoking. In addition, observational studies are important to investigate causes with a long latency period, such as carcinogenic effects of environmental exposures or drugs (49). Thus, possible adverse long-term effects of masks, i.e., comparable to the environmental hazards, appeared to be particularly detectable through observational studies.

The article "Physio-metabolic and clinical consequences of wearing face masks—Systematic review with meta-analysis and comprehensive evaluation" was retracted in 2023. Reasons: concerns about the data; concerns about the results or conclusions.

Finally, the random statistical control calculations of our results were performed for quality assurance *via* the R software (R Foundation for Statistical Computing, Vienna, Austria, version 4.0.1) and packages metafor, dmetar, meta (36). Knapp-Hartung adjustments to control for the uncertainty in the estimate of the between-study heterogeneity were used in these calculations which are controversial as they result in wider confidence intervals and are also suspected to be anti-conservative even though the effects are very homogeneous (36).

## Results

### General findings

#### Literature characteristics

Of the 2,168 screened records, 54 studies were included for qualitative analysis (see extraction tables, Table 1) and 37 for statistical meta-analysis (Figure 1). Among the 54 studies, 23 were intervention studies, and 31 were observational studies. The 23 intervention studies consisted of 14 randomized controlled trials (RCTs) and nine non-randomized controlled trials (nRCTs). Of the 31 observational studies, 17 works raised measured values, and 14 were questionnaire studies.

**Table 1A:** **(A–C)** Overview of 54 included studies. **(A)** Randomized controlled trials, **(B)** non-randomized controlled trials, and **(C)** observational studies.

**References**	**Study design**	**Intervention/control**	**Sample size**	**Time**	**Outcomes**
**(A) Included 14 randomized controlled trials**					
Bertoli et al. (50)	Randomized, two-period cross-over self-control trial	Wearing N95 respirator vs. no facemask during indirect calorimetry	*N* = 10	5 min	oxygen consumption (VO_2_), carbon dioxide production (VCO_2_), and Resting Energy Expenditure (REE)
Butz (51)	Blinded, randomized cross over study	Wearing two types of surgical masks vs. no mask	*N* = 15	30 min	CO_2_ under masks, PtCO_2_ (partial transcutaneous CO_2_ pressure) while wearing masks for 30 min, HR, RR (respiratory rate), and SpO_2_
Dirol et al. (52)	Prospective randomized cross-over study	Six-minutes walking test (6 MWT) with and without surgical mask. Mask-discomfort questionnaire was applied before and after 6 MWT with the mask	*N* = 100	6 min	RR, HR, SpO_2_, EtCO_2_, and discomfort questionnaire
Fikenzer et al. (53)	Prospective cross-over study	Wearing no mask (nm) vs. surgical mask (sm) vs. FFP2/N95 mask (ffpm), cardiopulmonary and metabolic responses monitored by ergo-spirometry and impedance cardiography	*N* = 12	10 min	FVC (forced vital capacity), FEV1 (forced expiratory volume in 1 s), Tiffenau index, peak expiratory flow (PEF), HR, stroke volume, cardiac output, arterio-venous oxygen content difference, systolic blood pressure (SBP), diastolic blood pressure (DBP), ventilation in liters/minute (VE), RR, tidal volume (VT), pH, partial pressure of carbon dioxide (PaCO_2_), partial pressure of oxygen (PaO_2_), lactate Pmax, Pmax/kg, VO_2_max/kg, heart rate recovery (HRR): HRR-1 min, HRR-5 min. Discomforts (VAS): humid, hot, breath resistance, itchy, tight, salty, unfit, odor, fatigue, and overall discomfort.
Georgi et al. (54)	Prospective randomized cross-over study	Wearing no mask (nm) vs. community vs. surgical mask vs. FFP2/N95 mask (treadmill: baseline, 50, 75, and 100 W)	*N* = 24	9 min	HR, RR, SBP, DBP, PtCO_2_, SpO_2_, and main symptoms questionnaire
Goh et al. (55)	Randomized, two-period cross-over self-control trial	Wearing N95 respirator vs. wearing N95 respirator with microfan vs. wearing no facemask during common physical activities	*N* = 106	15 min	EtCO_2_, comfort level with visual analog scale (VAS)
Hua et al. (47)	Prospective randomized crossover trial	Two and 4 h after donning the masks, adverse reactions and perceived discomfort and non-compliance were measured.	*N* = 20	240 min	Skin parameters: Skin hydration, transepidermal water loss, erythema, pH, and sebum secretion
Kim et al. (56)	Randomized and self-control trial	Wearing N95 respirator (partly with exhalation valve) vs. wearing no facemask (NM) during a low-moderate work-rate (5.6 km/h)	*N* = 20	60 min	HR, RR, transcutaneous carbon dioxide, and SpO_2_
Kim et al. (57)	Randomized and two-period controlled trial	Wearing N95 respirator and no mask during 1 h of mixed sedentary activity and moderate exercise during pregnancy vs. non-pregnant women	*N* = 16 vs. 16	60 min	SBP, DBP, mean arterial pressure, HR, stroke volume, cardiac output, total peripheral resistance, RPE, SpO_2_, and PtCO_2_
Kim et al. (58)	Randomized and self-control trial	Wearing N95 respirator vs. wearing P100 respirator vs. wearing no mask during 1 h of treadmill exercise (5.6 km/h) in an environmental chamber (35°C, relative humidity 50%)	*N* = 12	60 min	Fit factor, rectal temperature, mean skin temperature, facial skin temperature under respirator, SpO_2_, PtCO2, HR, RR, breathing comfort, thermal sensation, and exertion (Borg scale)
Mapelli et al. (59)	interventional, prospective, randomized, double-blind, and cross-over study	Wearing no mask surgical mask or N95 mask and performing consecutive cardiopulmonary exercise tests (CPETs) at least 24 h apart but within 2 weeks	*N* = 12	10 min	Ventilation (VE), Oxygen intake VO_2_, VCO_2_ production, respiratory gases, exspiratory O_2_ (ETO_2_) and exspiratory CO_2_ (ETCO_2_), heart rate (HR), hemoglobin saturation (SaO_2_), blood pressure (DBP and SBD), dyspnea (Borg scale), spirometry, maximal inspiratory pressure (MIP), and maximal expiratory pressure (MEP)
Roberge et al. (60)	Randomized and two-period controlled trial	Wearing an N95 FFR during exercise and postural sedentary activities over a 1-h period on pregnant women vs. control	*N* = 22/22	60 min	Core temperature, cheek temperature, abdominal temperature, HR, RR, RPE, and perceived heat (RHP)
Wong et al. (61)	Randomized and two-period self-controlled trial	Wearing a facemask vs. not wearing a facemask during graded treadmill (10% slope) walking at 4 km/h for 6 min	*N* = 23	6 min	HR and RPE
Zhang et al. (62)	Prospective randomized cross-over study	Exercises (cycle ergometer) with and without surgical masks (mask-on and mask-off) were analyzed	*N* = 71	8 min	Test duration, maximum power, RPE score, Borg dyspnea scale, Oxygen consumption (V. O_2_), carbon dioxide production (V.CO_2_), metabolic equivalent (MET), respiratory exchange rate (RER), and percentage of oxygen uptake at anaerobic threshold (AT) in predicted maximal oxygen uptake, inspiratory time (Ti), expiratory time (Te), RR, VT, V_E_, end-tidal oxygen partial pressure (EtO_2_), EtCO_2_, oxygen ventilation equivalent (VE/V.O2), and carbon dioxide equivalent (V_E_/VCO_2_)

The article "Physio-metabolic and clinical consequences of wearing face masks—Systematic review with meta-analysis and comprehensive evaluation" was retracted in 2023. Reasons: concerns about the data; concerns about the results or conclusions.

**Table 1B:** Included nine non-randomized controlled trials.

**References**	**Study design**	**Intervention/control**	**Sample size**	**Time**	**Outcomes**
Bharatendu et al. (63)	Cross-sectional self-control trial	Wearing N95 respirator vs. no facemask	*N* = 154	5 min	Mean flow velocity (MFV), pulsatility-index, end-tidal carbon dioxide partial pressure (EtCO_2_)
Coniam (64)	Two-period controlled trial	Wearing surgical masks (WM) vs. no facemask (NM) during oral examination	*N* = 186	10 min	Pronunciation, vocabulary, grammar, comprehensibility, and audibility
Epstein et al. (65)	Multiple cross-over, self-control trial	Wearing N95 respirator vs. wearing surgical mask vs. no facemask during maximal exercise test	*N* = 16	18 min	HR, RR, SpO_2_, rated perceived exertion (RPE), and end-tidal carbon dioxide (EtCO_2_)
Lee and Wang (66)	Two-period self-controlled trial	Wearing N95 respirator vs. no facemask during rhinomanometry	*N* = 14	30 sec	Inspiration breathing resistance increment, expiration breathing resistance increment, breathing volume decrement
Roberge et al. (67)	Multiple cross-over and self-control trial	Wearing an N95 FFR vs. N95 FFR with exhalation valve vs. no mask during 1-h treadmill walking sessions, at 1.7 miles/h and at 2.5 miles/h	*N* = 10	60 min	FFR dead space gases, CO_2_ saturation, O_2_ saturation, RR, VT, VE, and HR
Roberge et al. (68)	Two-period self-control trial	Wearing a surgical mask for 1 h during treadmill exercise at 5.6 km/h vs. the same exercise with no mask	*N* = 20	60 min	Core temperature, cheek temperature, abdominal temperature, HR, RR, RPE, and Perceived heat (RHP)
Scarano et al. (69)	Two-period self-controlled trial	Wearing a surgical mask for 1 h vs. wearing N95 respirator for 1 h vs. baseline	*N* = 20	60 min	Humidity, heat, breathing difficulty, discomfort, mask touching, and perioral temperature
Shenal et al. (70)	Multiple cross-over self-controlled field trial	Wearing one of seven respirators or medical mask during an 8-h working period vs. no mask	*N* = 27	480 min	Discomfort and RPE
Tong et al. (71)	Two-period self-controlled trial	Breathing through N95 mask materials during rest and exercise of predetermined intensity vs. breathing ambient air	*N* = 19	50 min	Oxygen consumption (VO_2_), carbon dioxide production (VCO_2_), VT, RR, VE, expired oxygen (FeO_2_), expired carbon dioxide (FeCO_2_), inspired oxygen (FiO_2_), and inspired carbon dioxide (FiCO_2_)

The article "Physio-metabolic and clinical consequences of wearing face masks—Systematic review with meta-analysis and comprehensive evaluation" was retracted in 2023. Reasons: concerns about the data; concerns about the results or conclusions.

**Table 1C:** Included 31 observational studies.

**References**	**Study design**	**Intervention/control**	**Sample size**	**Time**	**Outcomes**
Beder et al. (72)	Longitudinal and prospective observational study	Wearing surgical mask during major operations vs. baseline	*N* = 53	60–240 min	SpO_2_ (oxygen saturation), HR (heart rate)
Choudhury et al. (73)	Prospective cohort study	Wearing N95 respirator during light work vs. wearing full PPE during heavy work vs. baseline	*N* = 75	240 min	HR, SpO_2_, Perfusion Index (PI), RPE (rated perceived exertion), and modified Borg scale for dyspnoea
Foo et al. (74)	Survey study	Self-administered questionnaire healthcare workers	*N* = 322	480 min	Prevalence of adverse skin reactions
Forgie et al. (75)	Cross-sectional survey study	Self-administered questionnaire	*N* = 80	Not given	Mask/shield preference Mask results, shield results
Heider et al. (76)	Cross-sectional survey study	Validated Voice Handicap Index (VHI)-10 questionnaire and self-administered questionnaire	*N* = 221	480 min	Vocal symptoms, Spanish validated Voice Handicap Index (VHI)-10 questionnaire
Islam et al. (77)	Prospective cross-over self-control study	Wearing FFP2 (N95) mask for 30 min under sitting condition in an air-conditioned room	*N* = 10	30 min	Saha Institute of Nuclear Physics, Department of Atomic Energy, Government of India
Jafari et al. (78)	Cross-sectional study	Self-administered questionnaire, SpO_2_, HR, and venous blood samples	*N* = 243	240 min	RR, HR, SpO_2_, and salivary metabolic signature
Kao et al. (79)	Prospective observational study	Wearing N95 respirator during hemodialysis vs. baseline	*N* = 39	240 min	HR, RR, systolic blood pressure (SBP), diastolic blood pressure (DBP), PaO_2_, and PaCO_2_ discomfort rates
Klimek et al. (80)	Cross-sectional survey study	Visual Analog Scales (VAS) to document patient-reported symptoms and diagnostic findings	*N* = 46	120 min	Visual Analog Scales (VAS) to document patient-reported symptoms of rhinitis or rhinorrhea. mucosal irritation, secretion and edema in nasal endoscopy was graded
Kyung et al. (81)	Prospective panel study	Wearing N95 respirator during 6-min walking test vs. baseline	*N* = 97	6 min	SBP, DBP, HR, RR, EtCO_2_, and SpO_2_
Lan et al. (82)	Cross-sectional survey study	Self-administered questionnaire	*N* = 542	360 min	Prevalence of adverse skin reactions
Li et al. (83)	Prospective observational study	Exercise on a treadmill while wearing the protective facemasks	*N* = 10	100 min	HR, temperature and humidity (outside and inside the facemask), SBP, DBP, mask outer humidity, face microclimate humidity, chest microclimate humidity, mask outside temperature, face microclimate temperature, face skin temperature, chest microclimate temperature, subjective sensations: humidity, heat, breath resistance, itching, tightness, feeling salty, feeling unfit, feeling odorous, fatigue, and overall discomfort
Lim et al. (84)	Survey study	Self-administered questionnaire	*N* = 212	240 min	Prevalence of headaches
Luckman et al. (85)	Survey study using online experimental setting	Self-administered questionnaire and experimental online setting	*N* = 400	Not given	Risk compensation with reduced physical distancing (standing, sitting, and walking)
Matusiak et al. (86)	Cross-sectional survey study	Self-administered questionnaire	*N* = 876	Not given	Difficulty in breathing, warming/sweating glasses misting up, slurred speech, and itch
Mo (87)	Retrospective observation cross over cohort study	Wearing surgical mask vs. not wearing: compare to former hospitalizations. Including criteria: Patients who were hospitalized three or more times and at least two times before mask mandates	*N* = 23	7 min	Vital signs: temperature, HR, RR, SBP, DBP, serum and blood gas analysis, inpatient days. Clinical parameters, including ion concentration of serum, vital signs, inflammation markers, and artery blood gas.
Naylor et al. (88)	Survey study	Self-administered online questionnaires.	*N* = 129	Not given	Effects of certain aspects of lockdown, including face masks, social distancing, and video calling, on participants behavior, emotions, hearing performance, practical issues, and tinnitus.
Ong et al. (89)	Cross-sectional survey study	Self-administered questionnaire.	*N* = 158	360 min	PPE usage patterns, occupation, underlying comorbidities
Park et al. (90)	Prospective cohort study	Wearing KF94 respirator for 6 h vs. baseline	*N* = 21	360 min	Skin temperature increase, skin redness, skin hydration, sebum level, skin elasticity, and trans-epidermal water loss
Pifarré et al. (91)	Prospective trial	No mask baseline vs. mask baseline. Subjects wearing a mask immediately after a 21-flex test performed the Ruffier protocol	*N* = 8	5–7 min	PaO_2_, PaCO_2_, SpO_2_, and HR
Prousa (92)	Cross-sectional survey study	Self-administered questionnaire	*N* = 1,010	Not given	Wearing time, discomfort stress, tricks, psychovegetative complaints, positive feelings, aggression, and depression
Ramirez-Moreno et al. (93)	Cross-sectional study in healthcare workers	Self-administered questionnaire	*N* = 306	420 min	Work type, type of face mask, number of hours worn per day (SD). pre-existing headache, comorbidity, other symptoms, Sleep disturbance, loss of concentration, irritability, photophobia, sonophobia, and sickness/vomiting
Rebmann et al. (94)	Multiple cross-over and self-control trial	Wearing only an N95 or an N95 with mask overlay for a 12-h shift vs. baseline	*N* = 10	720 h	SBP, DBP, CO_2_ saturation, SpO_2_, HR, headache, nausea, light-headedness, and visual challenge
Rosner (95)	Cross-sectional study in healthcare workers	Self-administered questionnaire	*N* = 343	360 min	Acne, headache, skin breakdown (nose bridge, cheeks, chin, behind ears), and impaired cognition
Sukul et al. (26)	Two-period controlled trial	Wearing a surgical or N95 mask during rest (young to mid-aged adults were measured for 30 min and older adults were measured for 15 min)	*N* = 30	15–30 min	Exhaled breath profiles within mask space by high-resolution real-time mass-spectrometry (PTR-ToF-MS): Aldehydes, hemiterpene, organosulfur, short-chain fatty acids, alcohols, ketone, aromatics, nitrile, and monoterpene. Hemodynamic parameters: SpO_2_, PETCO_2_, HR, RR, SBP, DBP, cardiac ouput, exhaled oxygen, and humidity.
Szczesniak et al. (96)	Survey study	Self-administered online questionnaire After mask restrictions vs. before mask restrictions	*N* = 1,476 vs. 564	Not given	Employment status, place of residence, worktime per week, somatic symptoms, anxiety and insomnia, social dysfunction, and depression
Szepietowski et al. (97)	Survey study	Self-administered online questionnaire	*N* = 2,307	Not given	Itch, mask types used, and duration of mask use per day
Techasatian et al. (98)	Prospective cross-sectional survey study	Self-administered questionnaire	*N* = 833	480 min	Factors associated with adverse skin reaction, risk factors for adverse skin reaction, differences between HCW, and non-HCW
Thomas et al. (99)	Two-period controlled trial	Comparing the ability to accurately record 20 randomized aviation terms transmitted over the radio by a helicopter emergency medical services (HEMS) pilot wearing a surgical facemask and six different N95s with and without the aircraft engine operating	*N* = 3	Not given	Accurately record 20 terms transmitted over the radio by (HEMS) pilot wearing a surgical facemask or N95 mask
Toprak and Bulut (100)	Prospective observational study	surgical vs. N-95 mask *n* = 149 vs. *n* = 148	*N* = 297	35 min	Maternal vital signs: SBP, DBP, HR, RR, fever centigrade, and SpO_2_
Tornero-Aguilera and Clemente-Suárez (101)	Two-period controlled trial	Wearing a surgical facemask vs. not wearing a facemask during 150 min university lessons	N=50	150 min	Mental fatigue perception, reaction time (ms) SpO_2_, mean RR (ms), mean HR (bpm) square root of the mean value of the sum of squared differences of all successive R-R intervals (RMSSD; ms), low frequency (LF) and high-frequency (HF) normalized units (n.u.), SD1 (ms), and SD2 (ms)

AT, anaerobic threshold; DBP, diastolic blood pressure; EtCO_2_, end-tidal CO_2_ partial pressure; ESRD, end stage renal disease; TEWL, trans-epidermal water loss; FEV1, forced expiratory volume in 1 s; FVC, forced vital capacity; HCW, health care worker; HD, hemodialyis; HR, heart rate; MEP, maximal expiratory pressure; TMET1, metabolic equivalent; MIP, maximal inspiratory pressure; PEF, peak expiratory flow; PetCO_2_, end-tidal carbon dioxide pressure; PetO_2_, end-tidal oxygen pressure; PI, perfusion index; PPE, personal protective equipment; PtCo_2_, partial transcutaneous CO_2_ pressure; RER, respiratory exchange ratio; RPE, rated perceived exertion; RR, respiratory rate; RR, respiratory rate; SaO_2_, hemoglobin oxygen saturation; SBP, systolic blood pressure; SpO_2_, oxygen saturation; Te, expiratory time; Ti, inspiratory time; Ttot, Inspiratory + expiratory time; TV, tidal volume; V·CO_2_, carbon dioxide production; V·O_2_, oxygen uptake; V_E_, ventilation in liters/min; VE, ventilation; VT, tidal volume.

The article "Physio-metabolic and clinical consequences of wearing face masks—Systematic review with meta-analysis and comprehensive evaluation" was retracted in 2023. Reasons: concerns about the data; concerns about the results or conclusions.

**Figure 1:** PRISMA flow chart of the systematic review. From initial 2168, fifty-four studies were later included in the qualitative synthesis. Finally, 37 studies were evaluated statistically in the meta-analysis (quantitative analysis).

#### Quality appraisal

The quality of the studies was not very homogeneous. The quality assessment identified some studies with low and average quality, which were excluded from the meta-analysis. We included only high-quality studies in our meta-analysis of RCTs and nRCTs. The quality of the included observational studies is predominantly good. Tables 2A–D summarizes the results of the quality appraisal of the included research papers.

**Table 2A:** Quality appraisal of randomized trials (Cochrane RoB tool++).

	**Selection bias**		**Performancebias**	**Detection bias**	**Attrition bias**	**Reporting bias**	
**References**	**1. Random sampling**	**2. Allocation blinding**	**3. Blinding for intervention**	**4. Evaluation blinding**	**5. Incomplete data**	**6. Selective reporting**	**7. Other bias**
Bertoli et al. (50)	LR	LR	HR	HR	LR	UC	LR
Butz (51)	LR	LR	HR	LR	UC	UC	UC
Dirol et al. (52)	LR	LR	HR	LR	LR	LR	LR
Fikenzer et al. (53)	LR	LR	HR	LR	LR	LR	LR
Georgi et al. (54)	LR	LR	HR	LR	LR	UC	LR
Goh et al. (55)	LR	LR	HR	LR	LR	LR	LR
Hua et al. (47)	LR	LR	HR	LR	UC	UC	LR
Kim et al. (56)	HR	LR	HR	LR	LR	LR	LR
Kim et al. (57)	LR	LR	HR	LR	LR	UC	LR
Kim et al. (58)	LR	LR	HR	LR	LR	UC	LR
Mapelli et al. (59)	LR	LR	HR	LR	LR	UC	LR
Roberge et al. (60)	LR	LR	HR	LR	LR	UC	LR
Wong et al. (61)	LR	LR	HR	LR	LR	UC	LR
Zhang et al. (62)	LR	LR	HR	LR	LR	LR	LR

**(A)** Shows the quality analysis of RCTs with Cochrane RoB tool++. LR = low risk; HR = high risk; UC = Unclear.

**Table 2B:** Quality appraisal of non-randomized controlled trials (CASP checklist).

**References**	**1. Clear focus?**	**2. Appropriate methods?**	**3. Recruitment comprehensible? **	**4. Valid measurement of exposure? **	**5. Valid measurementof outcome?**	**6. Equality of groups?**	**7. Confounders taken intoaccount?**	**8. Sufficient size and significance of the effect? **	**9. Credibility of the results?**	**10. Transferability to other populations? clear focus? **	**11. Comparability with existing evidence? **
Bharatendu et al. (63)	Y	Y	Y	Y	UC	Y	Y	Y	UC	Y	UC
Coniam (64)	UC	N	Y	Y	Y	UC	UC	Y	Y	Y	UC
Epstein et al. (65)	Y	Y	Y	Y	Y	Y	UC	N	Y	Y	Y
Lee and Wang (66)	Y	Y	Y	Y	N	Y	Y	N	UC	Y	UC
Roberge et al. (68)	Y	Y	Y	Y	Y	Y	Y	Y	N	Y	Y
Roberge et al. (67)	Y	Y	Y	Y	Y	Y	Y	N	Y	Y	Y
Scarano et al. (69)	Y	Y	Y	Y	Y	Y	UC	Y	Y	Y	UC
Shenal et al. (70)	Y	Y	Y	Y	Y	Y	Y	Y	Y	Y	UC
Tong et al. (71)	Y	Y	Y	Y	N	Y	Y	Y	Y	Y	UC

**(B)** Lists the results of the quality analysis of nRCTs with CASP checklist, Y = yes, N = no, UC = unclear.

**Table 2C:** Quality appraisal of the observational studies (CASP checklist).

**References**	**1. Clear focus?**	**2. Appropriate methods?**	**3. Recruitment comprehensible?**	**4. Valid measurement of exposure?**	**5. Valid measurement of outcome?**	**6. Equality of groups?**	**7. Confounders taken into account?**	**8. Sufficient size and significanceof the effect?**	**9. Credibility of the results?**	**10. Transferability to other populations?clear focus?**	**11. Comparability with existing evidence?**
Beder et al. (72)	Y	Y	N	Y	Y	UC	N	Y	Y	Y	Y
Choudhury et al. (73)	Y	Y	Y	Y	Y	N	Y	Y	Y	N	N
Islam et al. (77)	Y	Y	Y	Y	Y	Y	UC	Y	UC	Y	Y
Jafari et al. (78)	Y	Y	Y	Y	Y	Y	UC	Y	Y	N	UC
Kao et al. (79)	Y	Y	Y	Y	Y	Y	Y	Y	Y	N	UC
Klimek et al. (80)	Y	Y	Y	Y	Y	Y	UC	Y	Y	Y	UC
Kyung et al. (81)	Y	Y	Y	Y	Y	Y	Y	Y	Y	N	UC
Li et al. (83)	Y	Y	Y	Y	Y	Y	Y	UC	Y	Y	UC
Luckman et al. (85)	Y	UC	N	Y	Y	Y	Y	Y	Y	Y	UC
Mo (87)	Y	Y	Y	Y	Y	UC	UC	Y	Y	Y	Y
Park et al. (90)	Y	Y	Y	Y	Y	Y	N	Y	Y	Y	UC
Pifarré et al. (91)	Y	Y	Y	Y	Y	Y	Y	Y	Y	Y	UC
Rebmann et al. (94)	Y	Y	Y	Y	Y	Y	N	N	Y	N	Y
Sukul et al. (26)	Y	Y	Y	Y	Y	Y	Y	Y	Y	Y	UC
Thomas et al. (99)	Y	Y	Y	Y	Y	N	Y	Y	Y	Y	UC
Toprak and Bulut (100)	Y	Y	Y	Y	Y	UC	N	Y	Y	N	Y
Tornero-Aguilera and Clemente-Suárez (101)	Y	Y	Y	Y	Y	Y	N	Y	Y	Y	Y

**(C)** Is on the quality analysis of observational (non-questionnaire) studies with CASP checklist, Y = yes, N = no, UC = unclear.

The article "Physio-metabolic and clinical consequences of wearing face masks—Systematic review with meta-analysis and comprehensive evaluation" was retracted in 2023. Reasons: concerns about the data; concerns about the results or conclusions.

**Table 2D:** Quality appraisal of the questionnaire studies (CASP checklist).

	**Study design **	**Validity and reliability**		**Questionnaire quality**		**Questionnaire design**		**Sample**	**Distribution and response**			**Analysis**	**Results**			**Summary andrecommendation**	
**References**	**Was a questionnaire study an appropriate method? **	**Are the results valid andrealistic?**	**Does the questionnaire used provide reliable results? **	**Were sample questions provided? **	**Are the questions formulated in a clear and understandable way? **	**Details on how the questionnaire was prepared? **	**Was the questionnaire prepared in an appropriate manner? **	**Was the sample sufficiently large and representative? **	**Was information provided on how the questionnaire was made available? **	**Was information provided on response rates and exclusion criteria? **	**Was potential responsebias discussed?**	**Were the results analyzed appropriately? **	**Were all relevant results published? **	**Were both significant and non-significant results published? **	**Were results adequately interpreted? **	**Does the summary reflect the results of the study? **	**Were the results placed in context with existing literature? **
Foo et al. (74)	Y	Y	UC	N	UC	N	UC	Y	Y	Y	N	Y	Y	Y	Y	Y	Y
Forgie et al. (75)	Y	Y	Y	Y	Y	Y	Y	Y	Y	Y	N	UC	Y	N	Y	Y	Y
Heider et al. (76)	Y	Y	Y	Y	Y	Y	Y	Y	Y	Y	Y	Y	Y	Y	Y	Y	Y
Lan et al. (82)	Y	Y	UC	N	UC	N	UC	Y	Y	Y	N	Y	Y	Y	Y	Y	Y
Lim et al. (84)	Y	Y	UC	N	UC	N	UC	Y	N	Y	N	Y	Y	Y	Y	Y	Y
Matusiak et al. (86)	Y	Y	UC	N	UC	Y	Y	Y	Y	Y	N	Y	UC	Y	Y	Y	Y
Naylor et al. (88)	Y	Y	Y	Y	Y	Y	Y	Y	Y	Y	Y	Y	Y	Y	Y	Y	N
Ong et al. (89)	Y	Y	UC	N	UC	N	UC	Y	Y	Y	N	Y	Y	Y	Y	Y	Y
Prousa (92)	Y	N	Y	Y	Y	Y	Y	N	Y	N	N	Y	Y	Y	N	Y	UC
Ramirez-Moreno et al. (93)	Y	Y	UC	N	UC	Y	Y	Y	Y	Y	N	Y	Y	Y	Y	Y	Y
Rosner (95)	Y	Y	UC	N	UC	N	UC	Y	Y	N	N	Y	Y	Y	Y	Y	Y
Szczesniak et al. (96)	Y	N	UC	N	UC	N	UC	Y	Y	N	N	Y	UC	N	N	Y	Y
Szepietowski et al. (97)	Y	Y	UC	N	UC	Y	Y	Y	Y	N	N	Y	Y	Y	Y	Y	Y
Techasatian et al. (98)	Y	Y	UC	N	UC	N	UC	Y	Y	N	N	Y	Y	Y	Y	Y	Y

**(D)** Documents the quality analysis of the questionnaire studies using the CASP checklist, Y = yes, N = no, UC = unclear.

The article "Physio-metabolic and clinical consequences of wearing face masks—Systematic review with meta-analysis and comprehensive evaluation" was retracted in 2023. Reasons: concerns about the data; concerns about the results or conclusions.

#### Mask type

Of the 37 meta-analytically evaluated studies, 31 examined the N95 mask, 19 the surgical mask with one not reporting on the specific type of mask due to the predominantly psychological research topic. There were 14 Studies evaluating both mask types (surgical and N95) and we compared the results in a separate meta-analysis (see below, Meta-analysis of N95 mask vs. surgical mask).

#### Participants and time

In order to conduct the meta-analysis 8,641 subjects were included, totaling 22,127 individual measurements/surveys.

This population consisted of young (age = 34.8 ± 12.5) and predominantly female subjects (*m* = 2,482, *f* = 6,159).

Physiological, physical, and biochemical data was used in the meta-analyses comprising of 934 participants and 3,765 experimental measurements.

The pooled prevalence data was drawn from a study population of *n* = 8,128 and included 17,383 data entries.

Most of the 37 studies, evaluated in meta-analyses included healthy participants. Twelve studies were conducted in health care workers (32%).

Two studies (5%) included chronic obstructive pulmonary disease (COPD), one study on hemodialysis patients, another study included children (3%) and four studies involved pregnant women (11%).

The median experimental time of the studies included in the meta-analyses (mostly controlled trials) on physiological, physical, and chemical face mask effects was 18 min with an interquartile range (IQR) of 50 min (min.: 6 min, max.: 360 min). There was a major variation in mask wearing durations with several outliers leading to a large standard deviation (mean of 45.8 min with a standard deviation of 69.9 min). Therefore, the mean was not an appropriate parameter to characterize this distribution).

The study with the longest experimental duration (360 min, observational) included only 21 healthy participants, which corresponds to 2.2% of the total population studied (*n* = 934).

Interestingly, the studies on symptoms (including many observational studies) had significantly longer observation times and a mean of 263.8 ± 170.3 min (median 240, IQR 180) in a total of *n* = 8,128 participants.

#### Qualitative evaluation

Of the 54 included studies, 51 reported numerous adverse mask effects across multiple clinical disciplines, as already compiled in a previous scoping review (14). Also 14 of the 17 studies, which were not included in the meta-analysis reported those numerous mask effects.

Overall, our systematic review found mask related symptoms that can be classified under the previously described Mask-Induced Exhaustion Syndrome (MIES) (14), with typical changes and symptoms that are often observed in combination.

The article "Physio-metabolic and clinical consequences of wearing face masks—Systematic review with meta-analysis and comprehensive evaluation" was retracted in 2023. Reasons: concerns about the data; concerns about the results or conclusions.

Among the included 54 studies (Table 1), we detected and compiled reports on frequently statistically significant physiological and psychological changes (*p* < 0.05) belonging to the MIES such as:

- *increase in breathing dead space volume* (60, 65).
- *increase in breathing resistance* (53, 59, 66, 67, 83).
- *increase in blood carbon dioxide* (26, 51–58, 60, 62, 63, 65, 68, 71, 81, 87, 91, 94).
- *decrease in blood oxygen saturation* (26, 52–54, 57–60, 62, 67, 71, 72, 79, 81, 91, 94, 100, 101).
- *increase in heart rate* (26, 52, 56, 57, 60, 61, 67, 68, 72, 81, 83, 94, 100, 101).
- *decrease in cardiopulmonary capacity* (53, 59, 62).
- *changes in respiratory rate* (52–54, 56, 59, 60, 62, 68, 79, 81, 100).
- *shortness of breath and difficulty breathing* (47, 52–54, 58, 68, 69, 73, 79, 81, 83, 86, 87, 92, 94).
- *headache* (54, 63, 73, 78, 82, 84, 89, 92–95).
- *dizziness* (54, 79, 81).
- *feeling hot and clammy* (52, 53, 58, 60, 68, 69, 83, 86).
- *decreased ability to concentrate* (101).
- *decreased ability to think* (81, 94, 95, 101).
- *drowsiness* (95).
- *impaired skin barrier function* (47, 74, 95).
- *itching* (47, 52, 53, 74, 80, 82, 83, 86, 97, 98).
- *acne, skin lesions and irritation* (47, 68, 74, 81, 82, 86, 95, 98).
- *false sense of security* (85, 96).
- *overall perceived fatigue and exhaustion* (52–54, 57–62, 68, 70, 71, 73, 79, 83, 94).

Moreover, we could objectify additional symptoms of the MIES as follows:

- *decrease in ventilation* (53, 59, 62).
- *increase in blood pressure* (26, 52, 53, 59, 62, 81, 83, 87, 100).
- *increase of measured temperature of the skin under the mask* (58, 68, 69, 90).
- *increase of measured humidity of the air under the mask* (58, 69, 90).
- c*ommunication disturbance* (86, 88, 94, 95, 99).
- v*oice disorder* (76, 86).
- *perceived discomfort* (47, 52, 53, 69).
- *increased anxiety* (75, 88, 92).
- *increased mood swings or depressive mood* (75, 76, 88, 92).

and:

- *changes in microbial metabolism (lower gut and oral)* (26, 77).

However, three studies (6% of the included papers) describe the absence of adverse or even positive mask effects (50, 64, 96).

### Results of the meta-analysis

In the meta-analytic evaluation, we found biochemical, physiological, physical, and perceptual symptoms with face mask use. We were also able to meta-analyze the pooled prevalence of symptoms. These results are presented in detail below.

### Meta-analysis of biochemical effects of face masks

#### SpO_2_ and face masks

The results are summarized in Figure 2A.

The article "Physio-metabolic and clinical consequences of wearing face masks—Systematic review with meta-analysis and comprehensive evaluation" was retracted in 2023. Reasons: concerns about the data; concerns about the results or conclusions.

**Figure 2:** Forest **(left)** and funnel plots **(right)** of meta-analysis of blood oxygenation and blood carbon dioxide outcomes while wearing a face mask. All face mask types are initially considered together, later subgroups (surgical and N95) are evaluated. If studies examine two different mask types in parallel, the corresponding studies are marked: □ = surgical mask ■ = N95 mask. **(A)** Blood oxygen is significantly lowered in mask use. In the subgroup analysis this could also be found for N95 mask use. From the pooled analysis, it seems, that N95 mask may be responsible for a larger SpO_2_ drop than surgical masks. In studies evaluating both conditions (surgical and N95 mask) the N95 mask yielded always lower O_2_-values than the surgical masks. **(B)** In the pooled analysis, blood carbon dioxide (PtCO_2_, ETCO_2_, and PaCO_2_) is significantly elevated in mask use. This could be found for general mask use and in the subgroup analysis for surgical mask, and also for N95 mask use. In studies evaluating both conditions (surgical and N95 mask) the N95 mask yielded always higher CO_2_-values than the surgical masks.

In a pooled analysis, blood oxygen saturation resulted significantly lowered during mask use. This could be found for general mask use (*p* = 0.0004, SMD = −0.24, 95% CI −0.38 to −0.11, *Z* = 3.53, *I*^2^ = 0%). The Eggers' test did not indicate the presence of funnel plot asymmetry [*t*_(df = 11)_ = −0.70, *p* = 0.50]. This was also confirmed in the subgroup analysis for N95 mask use (*p* = 0.001, SMD = −0.3, 95% CI −0.49 to −0.12, *Z* = 3.19, *I*^2^ = 0%), but not for surgical mask use [*p* = 0.08, SMD = −0.17, 95% CI (−0.37; 0.02), *Z* = 1.77, *I*^2^ = 0%]. However, seven of nine studies in the N95 mask meta-analysis were presumably because of the limited sample size. From the pooled analysis, it seems that N95 mask use may be responsible for a larger SpO_2_ drop than surgical masks.

In a separate meta-analysis of pre-post studies an equally significant drop in SpO_2_ was found when using a mask (*p* = 0.0001, SMD = −1.24, 95% CI −1.87 to −0.61, *Z* = 3.87, *I*^2^ = 80%) and especially in the subgroup of N95 masks (*p* = 0.02, SMD = −1.24, 95% CI −2.26 to −0.22, *Z* = 2.37, *I*^2^ = 89%), yet with a high heterogeneity.

#### Blood CO_2_ content and face masks

The results are summarized in Figure 2B.

In a pooled analysis, blood carbon dioxide content was found to be significantly elevated in mask use. This was found for general mask use (*p* = 0.0001, SMD = 0.64, 95% CI 0.31 to 0.96, *Z* = 3.86, *I*^2^ = 81%). The Eggers' test did not indicate the presence of funnel plot asymmetry [*t*_(df = 11)_ = −0.87, *p* = 0.40]. This was also confirmed for N95 mask use (*p* = 0.003, SMD = 0.78, 95% CI 0.28 to 1.29, *Z* = 3.02, *I*^2^ = 84%) and also for surgical mask use (*p* < 0.001, SMD = 0.42, 95% CI 0.24 to 0.59, *Z* = 4.65, *I*^2^ = 0%).

The article "Physio-metabolic and clinical consequences of wearing face masks—Systematic review with meta-analysis and comprehensive evaluation" was retracted in 2023. Reasons: concerns about the data; concerns about the results or conclusions.

There was no significant difference between the pooled effect sizes of N95 and surgical masks [*Q*_(df = 1)_ = 3.09, *p* = 0.08]. Further separate pooled evaluations were also carried out for PtCO_2_, ETCO_2_, and PaCO_2_, for each surgical and N95 masks with a significant increase in blood CO_2_ with predominantly low heterogeneity.

Even in a separate meta-analysis of pre-post studies with high heterogeneity, a significant increase in blood carbon dioxide content was found when using a mask (*p* = 0.003, SMD = 1.44, 95% CI 0.49 to 2.39, *Z* = 2.97, *I*^2^ = 94%) and also in the subgroup of N95 masks (*p* = 0.02, SMD = 1.51, 95% CI 0.24 to 2.78, *Z* = 2.34, *I*^2^ = 96%).

Interestingly, 11 of 17 showed no statistically significant effect. The studies that showed statistically significant effects differed from those that showed no certain effects as they either included N95 and/or pregnant women or children. The study by Dirol et al. (52) is an exception but has a sample size of *n* = 100 for surgical masks. Apparently, it takes N95 masks and vulnerable populations or appropriately large samples in surgical masks to make the effects more quantifiable.

Predictably, in the surgical mask meta-analysis, studies with non-significant results were of small sample size, with a mean of *n* = 24 and a median of *n* = 14. The advantage of a meta-analysis is to combine several imprecise effects into a more precise overall effect (36).

### Meta-analysis of physiological effects of face masks

#### Ventilation (V_*E*_) in L/min and face masks

The results are summarized in Figure 3A.

**Figure 3:** Forest **(left)** and funnel plots **(right)** of meta-analysis of physiological respiratory outcomes while wearing a face mask. **(A)** Shows results for ventilation (V_E_), **(B)** for respiratory rate (RR). All face mask types are initially considered together, later subgroups (surgical and N95) are evaluated. If studies examine two different mask types in parallel, the corresponding studies are marked: □ = surgical mask ■ = N95 mask. **(A)** Breathing volume is significantly lowered in mask use in the pooled analysis. This could be found for general, for surgical, and N95 mask use. In studies evaluating both conditions (surgical and N95 mask) the N95 mask yielded always lower ventilation (V_E_) than the surgical masks. **(B)** No statistical difference could be found regarding respiratory rate in mask use in the pooled analysis, even in the subgroup analysis (not shown).

The article "Physio-metabolic and clinical consequences of wearing face masks—Systematic review with meta-analysis and comprehensive evaluation" was retracted in 2023. Reasons: concerns about the data; concerns about the results or conclusions.

Despite compensatory mechanisms, breathing volume (L/min) was significantly lowered during mask use in the pooled analysis.

This was not only verified for general mask use (*p* < 0.001, SMD = −0.72, *Z* = 5.36, 95% CI −0.99 to −0.46, *I*^2^ = 0%) in studies evaluated with an overall low heterogeneity (*I*^2^ = 0), but also for surgical (*p* < 0.001, SMD = −0,54, 95% CI −0.94 to −0.35, *Z* = 4.32, *I*^2^ = 0%) and N95 mask use (*p* = 0.0007, SMD = −1.06, 95% CI −1.68 to −0.45, *Z* = 3.39, *I*^2^ = 0%). Both studies had an overall low heterogeneity (*I*^2^ = 0).

On average, masks reduced respiratory minute volume by −19% according to our meta-analysis, and by as much as −24% for N95 masks; the difference between surgical and N95 masks was −10% respiratory minute volume.

#### Respiratory rate and face masks

The results are summarized in Figure 3B.

Interestingly, no statistical difference regarding respiratory rate was found in mask use in the pooled analysis.

Even in the subgroups containing N95 and surgical masks, no difference compared to the no mask condition could be found.

#### Systolic blood pressure and masks

The results are summarized in Figure 4A.

**Figure 4:** Forest **(left)** and funnel plots **(right)** of meta-analysis of the physiological cardiovascular outcomes systolic blood pressure (SBP) and heart rate (HR). All controlled intervention studies in which measurements were taken during physical activity with face masks were included (exclusion of rest situation and pre-post studies). All face masks types are initially considered together, later if possible subgroups (surgical and N95) are evaluated. If studies evaluate two different mask types in parallel, the corresponding studies are marked: □ = surgical mask ■ = N95 mask. **(A)** Systolic blood pressure is elevated in the mask condition and also for the subgroup of surgical mask. In studies evaluating both conditions (surgical and N95 mask) the N95 mask yielded always higher SBP than the surgical mask, however this effect was not statistically significant. **(B)** For the N95 mask condition a low significance for a slight increase in heart rate could be found. In studies evaluating both conditions (surgical and N95 mask) the N95 mask yielded always higher HR than the surgical mask, and this effect was statistically significant.

A significant elevation in systolic blood pressure was found for mask users with *p* = 0.02, SMD = 0.17, 95% CI 0.03 to 0.32, *Z* = 2.39 and *I*^2^ = 0% in the pooled analysis. It was a small effect and in nine out of 10 studies insignificant, including two with higher n in each case. The Eggers' test does not indicate the presence of funnel plot asymmetry [*t*_(df = 8)_, *p* = 0.27]. This was verified in the subgroup analysis for surgical masks (*p* = 0.02, SMD = 0.21, 95% CI 0.03 to 0.39, *Z* = 2.33, *I*^2^ = 0%). In studies evaluating both mask types (surgical and N95) the N95 mask always yielded a higher SBP than the surgical mask. However, this effect was not statistically significant. There was no significant difference between the pooled effect sizes of N95 and surgical masks [*Q*_(df = 1)_ = 0.98, *p* = 0.32].

The article "Physio-metabolic and clinical consequences of wearing face masks—Systematic review with meta-analysis and comprehensive evaluation" was retracted in 2023. Reasons: concerns about the data; concerns about the results or conclusions.

#### Heart rate and masks

The results are summarized in Figure 4B.

No statistically significant difference regarding the heart rate during mask use was found in the pooled analysis. The Eggers' test did not indicate the presence of funnel plot asymmetry [*t*_(df = 14)_, *p* = 0.94]. However, in the subgroup analysis containing surgical and N95 masks, only for the N95 mask condition a weak significance for a slight increase in heart rate could be found (*p* = 0.02, SMD = 0.22, 95% CI 0.03 to 0.41, *Z* = 2.30 and low heterogeneity of studies with *I*^2^ = 0). There was no significant difference between the pooled effect sizes of N95 and surgical masks [*Q*_(df = 1)_ = 1.26, *p* = 0.26].

### Meta-analysis of physical effects of face masks

#### Skin temperature and face masks

The results are summarized in Figure 5A.

**Figure 5:** Forest **(left)** and funnel plots **(right)** of meta-analysis of physical outcomes while wearing a face mask. **(A)** Shows results for temperature of skin, **(B)** for air humidity underneath the face mask. All mask types are initially considered together, later subgroups (surgical and N95) are evaluated. If studies examine two different mask types in parallel, the corresponding studies are marked: □ = surgical mask ■ = N95 mask. **(A)** Skin covered by mask has a significantly higher temperature during rest and activity. This could be found for general mask use and for N95 mask use but not for surgical mask use. In studies evaluating both conditions (surgical and N95 mask) the N95 mask yielded higher temperatures than the surgical mask, but this could not be analyzed further due to lack of further studies comparing both conditions. **(B)** The dead space covered by mask has a significantly higher air humidity in the pooled analysis.

Skin covered by mask had a significantly higher temperature during rest and activity. This could be found for general mask use (*p* = 0.005, SMD = 0.80, 95% CI 0.23 to 1.38, *Z* = 2.81. *I*^2^ = 72%), for N95 mask use (*p* = 0.02, SMD = 0.72, 95% CI 0.12 to 1.32, *Z* = 2.35, *I*^2^ = 55%), but not for surgical mask use (*p* = 0.21, SMD = 0.96, *Z* = 1.26, *I*^2^ = 90%).

The article "Physio-metabolic and clinical consequences of wearing face masks—Systematic review with meta-analysis and comprehensive evaluation" was retracted in 2023. Reasons: concerns about the data; concerns about the results or conclusions.

#### Humidity and face masks

The results are summarized in Figure 5B.

The dead space covered by mask had a significantly higher humidity in the pooled analysis.

This could be found for general mask use with *p* < 0.001, SMD = 2.24, 95% CI 1.32 to 3.17, *Z* = 4.75 and *I*^2^ = 50%.

### Meta-analysis of measured symptoms and sensations during face mask use

#### Discomfort and face masks

The results are summarized in Figure 6A.

**Figure 6:** Forest and funnel plots of meta-analysis of measured discomfort **(A)**, itch **(B)**, exertion **(C)**, shortness of breath **(D)**, perceived heat **(E)**, and humidity **(F)** during face mask use (VAS, Likert-scales or similar) in an evaluated population of *n* = 373. All face mask types are initially considered together, later subgroups (surgical and N95) are evaluated. If studies examine two different mask types in parallel, the corresponding studies are marked: □ = surgical mask ■ = N95 mask. **(A)** Perceived discomfort is significantly higher in face mask use in the pooled analysis. This could be found for general mask use, in the subgroup analysis for surgical-, and for N95 mask use. A pooled analysis comparing both conditions (surgical mask and N95 mask) resulted in statistically significant higher discomfort rates for the N95 mask than the surgical mask. **(B)** An overall significance for itching could be found for mask use. Also in N95 mask use the perceived itching was statistically significantly elevated according to the pooled subgroup analysis. **(C)** In studies evaluating both conditions (surgical and N95 mask) the N95 mask yielded always higher exertion rates than the surgical masks. **(D)** Perceived shortness of breath is significantly higher in mask use in the pooled analysis. **(E)** Perceived heat is significantly higher in the pooled analysis. **(F)** Perceived humidity is significantly higher in mask use. The subgroup analysis revealed a statistical significance for an increase in humidity perception using a surgical mask. In studies evaluating both conditions (surgical and N95 mask) the N95 mask yielded always higher humidity perception rates than the surgical mask. A pooled analysis resulted in a statistical significance for higher humidity perception in N95 masks than surgical masks.

Perceived discomfort was significantly higher in mask use during rest and activity in the pooled analysis.

This could be found for general mask use (*p* < 0.001, SMD = 1.16, 95% CI 0.58 to 1.73, *Z* = 3.94, *I*^2^ = 74%), for N95 mask use (*p* < 0.001, SMD = 1.98, 95% CI 1.37 to 2.59, *Z* = 6.34, *I*^2^ = 0%) as well as for surgical mask use (*p* < 0.001, SMD = 0.71, 95% CI 0.46 to 0.96, *Z* = 5.58, *I*^2^ = 0%).

The article "Physio-metabolic and clinical consequences of wearing face masks—Systematic review with meta-analysis and comprehensive evaluation" was retracted in 2023. Reasons: concerns about the data; concerns about the results or conclusions.

#### Itch and face masks

The results are summarized in Figure 6B.

In N95 mask use, the perceived itching was significantly elevated (*p* = 0.003, SMD = 2.65, 95% CI 1.21 to 4.09, *Z* = 3.6, *I*^2^ = 83%) during activity according to the pooled subgroup analysis.

#### Exertion and face masks

The results are summarized in Figure 6C.

Perceived exertion is significantly higher in mask use during activity in the pooled analysis.

This could be found for general mask use (*p* < 0.001, SMD = 0.90, 95% CI 0.58 to 1.23, *Z* = 5.31. *I*^2^ = 71%), for N95 mask use (*p* = 0.002, SDM = 1.19, 95% CI 0.43 to 1.95, *Z* = 3.06, *I*^2^ = 81%) as well as for surgical mask use (*p* < 0.001, SMD = 0.63, 95% CI 0.40 to 0.87, *Z* = 5.29, *I*^2^ = 24%). The Eggers' test indicates the presence of funnel plot asymmetry [*t*_(df = 10)_ = 2.68, *p* = 0.02]. For N95 mask use (*p* = 0.002, SDM = 1.19, *Z* = 3.06, *I*^2^ = 81%) and this result was confirmed for surgical mask use too (*p* < 0.001, SMD = 0.63, *Z* = 5.29, *I*^2^ = 24%). There was no significant difference between the pooled effect sizes of N95 and surgical masks [*Q*_(df = 1)_ = 1.97, *p* = 0.16].

#### Shortness of breath and face masks

The results are summarized in Figure 6D.

Perceived shortness of breath was significantly higher during mask use during activity in the pooled analysis (*p* = 0.006, SMD = 1.46, 95% CI 0.42 to 2.50, *Z* = 2.75, *I*^2^ = 86%).

#### Perceived heat and face masks

The results are summarized in Figure 6E.

Perceived heat is significantly higher during mask use with physical activity in the pooled analysis (*p* = 0.002, SMD = 0.70, 95%CI 0.28 to 1.13, *Z* = 3.27, *I*^2^ = 62%).

In the subgroup analysis containing surgical and N95 masks the heat perception was increased in both mask types, but only for the surgical mask condition a statistical significance for an increase in heat perception could be found (*p* = 0.008, SDM = 0.61, 95% CI 0.16 to 1.06, *Z* = 2.66, *I*^2^ = 50%).

#### Perceived humidity and face masks

The results are summarized in Figure 6F.

Perceived humidity was significantly higher in mask use during activity according to the pooled analysis (*p* = 0.002, SMD = 0.90, 95% CI 0.34 to 1.46, *Z* = 3.17, *I*^2^ = 53%).

The subgroup analysis containing surgical and N95 masks was completed merely for surgical masks due to lack of studies on N95 masks.

In the surgical mask subgroup a statistical significance for an increase in humidity perception could be found (*p* < 0.001, SMD = 0.63, 95% CI 0.36 to 0.90, *Z* = 4.6, *I*^2^ = 0).

### Meta-analysis of N95 mask vs. surgical mask

The results are summarized in Figures 7A–C.

**Figure 7:** Results comparing the N95 to the surgical mask in the meta-analysis. Forest **(left)** and funnel plots **(right)** of meta-analysis of diverse outcomes while wearing a N95 mask vs surgical mask are shown. **(A)** Depicts the biochemical, **(B)** the cardiorespiratory outcomes, and **(C)** the subjective sensations outcomes. N95 mask leads to measurably less favorable results compared to the surgical mask, significantly for oxygenation (decrease), heart rate (increase), discomfort and humidity (both increases). This trend was also evident for minute volume (decrease), CO_2_ and systolic blood pressure (both increases), but in those comparisons not statistically significant due to too few includable studies.

The article "Physio-metabolic and clinical consequences of wearing face masks—Systematic review with meta-analysis and comprehensive evaluation" was retracted in 2023. Reasons: concerns about the data; concerns about the results or conclusions.

The N95 mask leds to measurably worse effects compared to the surgical mask. The blood oxygenation was significantly decreased when using a N95 mask compared to a surgical mask with *p* = 0.003, SMD = −0.53, 95% CI −0.88 to −0.18, *Z* = 2.98, *I*^2^ = 37%. The heart rate (*p* = 0.01, SMD = 0.25, 95% CI 0.05 to 0.45, *Z* = 2.47, *I*^2^ = 0%), the perception of discomfort (*p* = 0.02, SMD = 3.07, 95% CI 0.52 to 5.61, *Z* = 2.36, *I*^2^ = 95%) and humidity (*p* = 0.02, SMD = 0.59, 95% CI 0.09 to 1.10, *Z* = 2.32, *I*^2^ = 0%) increased when the N95 mask was compared to the surgical mask. This trend was also evident for blood content of CO_2_, minute volume, exertion, heat, shortened breath, and systolic blood pressure, but was not statistically significant due to the limited available studies.

### Meta-analysis with pooled prevalence of symptoms during face mask use

The results are summarized in Figure 8.

**Figure 8:** Forest **(left)** and funnel plots **(right)** of meta-analysis of pooled symptom prevalence while wearing a face mask. Headache (62%), acne (38%), skin irritation (36%), shortness of breath (33%), heat (26%), itch (26%), voice disorder (23%), and dizziness (5%) while wearing a mask are significant in the evaluated population (*n* = 8,128).

Headache was the most frequent symptom among *n* = 2,525 subjects, with a prevalence of 62% for general mask use (*p* < 0.001, 95% CI 0.48 to 0.75), up to 70% with N95 masks (*p* < 0.001, 95% CI 0.52 to 0.88). Additionally, the prevalence of acne in *n* = 1,489 evaluated mask users was quite high, at 38% (*p* < 0.001, 95% CI 0.22 to 0.54), and skin irritation in *n* = 3,046 mask users had a similar prevalence of 36% (*p* < 0.001, 95% CI 0.24 to 0.49). Shortness of breath was highly prevalent in *n* = 2,134 general mask users, with 33% (*p* < 0.001, 95% CI 0.23 to 0.44), up to 37% for N95 (*p* = 0.01, 95% CI 0.07 to 0.67). Itching was also present in 26% of *n* = 5,000 subjects (*p* < 0.001, 95% CI 0.15 to 0.36), with a sharp difference between the 51% of N95 (*p* < 0.001, 95% CI 0.47 to 0.55) and the 17% of surgical masks (*p* < 0.001, 95% CI 0.09 to 0.26). These results were confirmed in control calculations using the R software. Furthermore, voice disorders, assessed in *n* = 1,097, were 23% prevalent (*p* = 0.03, 95% CI 0.02 to 0.43), although with high heterogeneity of the studies. Finally, dizziness had a prevalence of only 5% (*p* = 0.01, 95% CI 0.01 to 0.09), however it was investigated in only *n* = 153 subjects, therefore this finding requires further studies.

The article "Physio-metabolic and clinical consequences of wearing face masks—Systematic review with meta-analysis and comprehensive evaluation" was retracted in 2023. Reasons: concerns about the data; concerns about the results or conclusions.

## Discussion

Besides possibly providing protection against the transmission of pathogens, face masks undoubtedly impede natural breathing. Such respiratory impairments due to the “new-normal” lifestyle under the present global pandemic have imposed potential adverse effects on our usual external (airways, lungs) and internal (cellular) respiration, affecting a wide range of physio-metabolic processes within various organ systems and/or at cellular levels (14, 26). Ensuing consequences were eventually observed at the physical, psychological and social levels along with certain clinical symptoms in the individual human beings (14). In this systemic review, we applied meta-analysis and comprehensive evaluations of physio-metabolic, physical, psychological and clinical burdens of wearing face masks in the general population. Restricting breathing through face masks has turned out to be a fundamental, incisive intervention with possible negative effects on public health.

### Physio-metabolic burden of masks

Our meta-analysis clearly depicts that masks, and especially the N95 masks, significantly restrict O_2_ uptake and hinder CO_2_ release. Based on the meta-analytic effect sizes defined by Cohen (102), the effect size for CO_2_ retention (as per PtCO_2_, ETCO_2_, and PaCO_2_ outcomes) is medium for all mask types and is larger for N95 masks. The effect size for O_2_ uptake disturbance (as per SpO_2_ outcome) is relatively smaller but highly significant (*p* = 0.0004; Figures 2A, B, 9A). Such respiratory gas-exchange discrepancy can be attributed to the constantly increased dead space ventilation volume (14, 60, 65, 103, 104) (i.e., continuous rebreathing from the masks dead space volume) and breathing resistance (14, 53, 59, 66, 67, 83). Continuous CO_2_ rebreathing causes the right-shift of hemoglobin*-*O_2_ saturation curve. Since O_2_ and CO_2_ homeostasis influences diverse down-stream metabolic processes, corresponding changes toward clinically concerning directions may lead to unfavorable consequences such as transient hypoxemia and hypercarbia, increased breath humidity, and body temperature along with compromised physiological compensations etc.

The article "Physio-metabolic and clinical consequences of wearing face masks—Systematic review with meta-analysis and comprehensive evaluation" was retracted in 2023. Reasons: concerns about the data; concerns about the results or conclusions.

**Figure 9:** Summary of pooled meta-analytic evaluation of biochemical **(A)** and physical effects **(B)** during face mask use. The height of the bars reflects the SMD (standard mean difference), their error bars correspond to the confidence intervals. **(A)** For carbon dioxide rise in the blood there is a medium effect size of >0.5 and for oxygen drop a small effect size of >0.2 regarding the standard mean difference values thresholds according to Cohen (102). **(B)** For elevated Humidity and Temperature rise under the face mask there is a strong effect size of ≥0.8. The meta-analytical statistical data were as follows: Oxygen (SpO_2_): SMD −0.24, 95% CI −0.38 to −0.11, *Z* = 3.53, *p* = 0.0004; Carbon dioxide (PtCO_2_, ETCO_2_, and PaCO_2_): SMD +0.64, 95% CI 0.31 to 0.96, *Z* = 3.86, *p* = 0.0001; Humidity: SMD +2.24, 95% CI 1.32 to 3.17, *Z* = 4.75, *p* < 0.00001; Temperature: SMD +0.8, 95% CI 0.23 to 1.38, *Z* = 2.72, *p* = 0.008.

### Transient hypoxemia

A progressive decrease in SpO_2_ is observed with respect to the duration of wearing a mask (26, 52, 56, 58, 72, 73, 81, 91, 105). The decline in SpO_2_ levels confirmed in our systemic-review supports the onset and progression of oxidative stress (*via* significantly increased exhaled breath aldehydes—originating from lipid peroxidation) reported by Sukul et al. (26). Studies have shown that oxidative stress (under hypoxic conditions) can inhibit cell-mediated immune response (e.g., T-lymphocytes, TCR CD4 complex, etc.) to fight viral infections, which may gradually lead to immune suppression (106, 107). Arterial hypoxemia increases the level of the hypoxia inducible factor-1α (HIF-1α), which further inhibits T-cells and stimulates regulatory T-cells (107). This may set the stage for contracting any infection, including SARS-CoV-2 and making the consequences of that infection much more severe. In essence, masks may put wearers at an increased risk of infection and severity (106–108). A recent review (109) by Serebrovska et al. discusses a possible link between HIF-1α activation and cell entry of SARS-CoV-2. If the cell is already under oxidative stress, activation of HIF-1α may suppress important adaptive mechanisms e.g., autophagy or proteasomal proteolysis is leads to the induction of necrosis and excessive cytokine production. Sturrock et al. (110) demonstrated that the SARS-CoV-2 receptor (e.g., ACE2 and TMPRSS2) expression by primary type II alveolar epithelial cells increased significantly following exposure to hypoxic environments *in vivo* and *in vitro*. Furthermore, recent research has demonstrated that the cellular entry of SARS-CoV-2 also depends on many other receptor paths/routes (e.g., CD147, CD147—spike proteins etc.), mediated by HIF-1α upregulation (111–114). Therefore, the effect of even mild hypoxemia for an extended span may promote an infection risk along with metabolic stress e.g., due to altered pH *via* respiratory acidosis. In line with that, Sukul et al. (26) observed a significant decrease in exhaled volatile metabolites (e.g., organosulfur and short-chain fatty acids) originating from the lower gut microbiota during face mask use—indicating anaerobiosis, metabolic acidosis and possible immunosuppression. Even marginal local effects of masks on salivary metabolites in young and healthy adults have indicated alteration of microbial metabolic activity (77).

The article "Physio-metabolic and clinical consequences of wearing face masks—Systematic review with meta-analysis and comprehensive evaluation" was retracted in 2023. Reasons: concerns about the data; concerns about the results or conclusions.

The findings of Spira (16) from European data show that mask use correlates with increased morbidity and mortality, which could be due to the above-discussed possible processes. Moreover, prolonged hypoxic conditions and low oxygen levels pave the way for immunosuppression and inflammation, which may promote the growth, invasion and spread of cancers (114–116).

However, further experimental studies are needed to prove that hypoxemia under long-term mask use may result in quantifiable changes in HIF-1α and immunosuppression—especially in older adults, ill/comorbid and/or immunocompromised individuals.

### Transient hypercarbia

In line with the increased dead space ventilation and consistently decreasing SpO_2_ level, CO_2_ inhalation elevates progressively during the course of wearing a mask, causing transient hypercarbia (26, 52, 56, 58, 81, 91, 105). Very recent experimental data exist on CO_2_ concentrations of concern in the air breathed while wearing masks, especially in children (117, 118). Systemic CO_2_ concentration exerts an important influence on the intra- and extracellular pH. CO_2_ passes quickly through the cell membranes to form carbonic acid, which releases protons and in excess causes acidosis (119–121). With a prolonged CO_2_ burden the body uses the bones (CO_2_ storage) to regulate the blood pH: bicarbonate and a positive ion (Ca^2+^, K^+^, and Na^+^) are exchanged for H^+^. Accordingly, kidney and organ calcification were frequently seen in animal studies on low-level CO_2_ exposure (122, 123). Additionally, CO_2_ in relationship with chronic and/or intermittent long-term exposure might induce pathological states by favoring DNA alterations and inflammation (124, 125). Moreover, inflammation is reported to be caused by low-level CO_2_ exposure in humans and animals (125–129). Even slightly elevated CO_2_ induces higher levels of pro-inflammatory Interleukin-1β, a protein involved in regulating immune responses, which causes inflammation, vasoconstriction and vascular damage (128). In addition, carbon dioxide is also known as a trigger of oxidative stress caused by reactive oxygen species (ROS) (124) including oxidative damage to cellular DNA (124, 125).

The article "Physio-metabolic and clinical consequences of wearing face masks—Systematic review with meta-analysis and comprehensive evaluation" was retracted in 2023. Reasons: concerns about the data; concerns about the results or conclusions.

Altogether, the possible damaging mechanism of CO_2_ affecting tissues is based on the conditions of oxidative stress and acidosis with increased inflammation and apoptosis as described above (124, 126–131). In the long term, therefore, this could be possible during mask use even at blood-CO_2_ levels that do not reach the thresholds. In spontaneously breathing subjects in a sitting position, exhaled CO_2_ profiles mirror the endogenous isoprene exhalation (18, 132). Significant and progressively decreased breath isoprene recently observed in adults (26) indicates the deoxygenation driven sympathetic vasoconstriction in the peripheral compartments (133). Prolonged deoxygenation and CO_2_ re-breathing therefore, may eventually lead to pulmonary vasoconstriction that may hinder blood-CO_2_ levels to reach the thresholds. For instance, Sukul et al. also reported the presence of significant hyperventilation state in older adults aged ≥ 60 years before wearing a face mask for the participation in experiments. This indicates a compromised respiratory compensation of precedent mask use (which was obligatory due to pandemic regulations at that time) by these subjects.

### Physical burden of masks: Humidity and skin temperature

Together with the immune-inhibiting mechanisms mentioned above, we found some other possible deleterious mask effects that impede healthy natural breathing. The most prominent and extreme effect was found in the increase of air humidity and skin temperature within the dead space of the mask (Figures 5, 9B). Increased humidity and temperature can increase droplet and aerosol generation, which facilitate liquid penetration through the mask mesh. This not only increases the chance of microorganism (fungal and bacterial pathogens) growth on and in masks (134–136) causing increased risk for accumulation of fungal and bacterial pathogens (134, 136) including mucormycosis (137), but also leading to re-breathing of viruses that may be trapped and enriched within the moisturized mask meshwork. Therefore, these conditions within masks are favorable for pathogenic growth and are unfavorable for good/systemic microbiota i.e., individual specific. As a result, the isolation of people with masks for extended periods can attain conditions for new and individual specific strains formations/mutations of pathogens—to which other people in the environment will be susceptible and/or not immune. Additionally, the high concentration of microbiome in masks can be a potential source of infection for the population. The findings of Fögen (11) using data from the USA which shows that mask use correlates with an increased mortality (case fatality rate of COVID-19) could be due to these processes. This phenomenon could also explain the similar figures found by Spira (16) in the EU.

The article "Physio-metabolic and clinical consequences of wearing face masks—Systematic review with meta-analysis and comprehensive evaluation" was retracted in 2023. Reasons: concerns about the data; concerns about the results or conclusions.

### Compensatory physiological mechanisms

Our meta-analytically quantified CO_2_-rise and O_2_-depletion (Figures 2, 9A) with mask use certainly needs physiological compensations (Figures 3, 4, 10). Interestingly, the compensatory responses to mask wearing (e.g., rise in heart rate, changes in respiratory rate and/or minute ventilation etc.) was lower (absent or even reverse) than expected (122, 138, 139). In former human experiments with low level 1-2% CO_2_ exposure to breathing air – which corresponds to measured values during mask use (140)—an increased respiratory minute volume (V_E_) of >34% was detected (122). In contrast to that and according to our results under masks a significantly decreased V_E_ by −19% on an average and up to −24% under N95 masks occurs despite face mask driven CO_2_ exposure (140). V_E_ was even 10% lower for the N95 than for the surgical masks (Figure 3A). However, it appears to have no acute clinical impact in the short term and does not exceed normal values of SpO_2_ and systemic CO_2_ although these may become problematic in the long run. A compensatory higher arterial PaCO_2_ and bicarbonate levels execute the buffering of inhaled CO_2_. Interestingly, during chronic breathing of low CO_2_ concentrations (in the no-mask condition), due to compensatory mechanisms, e.g., lowered blood pH, increased respiratory rate and V_E_ (122) and an acclimatization occurs (122, 138, 139, 141, 142). In mask users, those compensatory mechanisms however seem to differ or get disturbed (e.g., no rise in respiratory rate, heart rate and simultaneous fall in V_E_). Health risks should be considered despite the mask related compensation attempts (140). During face mask use a rise in the arterial PaCO_2_ is possible in the long term (26, 52, 81, 91, 105). Although, PaCO_2_ generally remains at a sub-threshold level in healthy mask users (105, 138), concerning pathological changes can occur in older (>60 years) and sick people (26, 87).

**Figure 10:** Summary of pooled meta-analytic evaluation of cardiorespiratory effects during face mask use. The height of the bars reflects the SMD (standard mean difference), their error bars correspond to the confidence intervals. Clear effects for a decrease in ventilation and tidal volume are illustrated, no effect for respiratory rate and weak to low effect for increase in heart rate and systolic blood pressure. For ventilation there is a medium effect size of >0.5 with a small effect size of >0.2 for tidal volume of the standard mean difference values according to Cohen (102). The meta-analytical statistical data were as follows: Ventilation: SMD −0.72, 95% CI −0.99 to −0.46, *Z* = 5.36, *p* < 0.00001; Tidal volume: SMD −0.37, 95% CI −0.63 to −0.11, *Z* = 2.82, *p* = 0.005; Respiratory rate: SMD +0.01, 95% CI −0.29 to 0.30, *Z* = 0.08, *p* = 0.94; Heart rate: SMD +0.11, 95% CI −0.05 to 0.28, *Z* = 1.34, *p* = 0.18; Systolic blood pressure: SMD +0.17, 95% CI 0.03 to 0.32, *Z* = 2.39, *p* = 0.02.

The article "Physio-metabolic and clinical consequences of wearing face masks—Systematic review with meta-analysis and comprehensive evaluation" was retracted in 2023. Reasons: concerns about the data; concerns about the results or conclusions.

Our findings depicted an absence of typical compensatory reactions to transient hypercarbia thereby implying a suppression of a physiological response owing to the unusual conditions of wearing a mask. The reasons behind this phenomenon, i.e., the absence of a rise in the respiratory rate and ventilation, remain unclear. The simultaneous change in the adverse direction (CO_2_ rise and simultaneous O_2_ fall with concomitant dead space- and resistance enlargement caused by the mask) may be responsible for this. The drop in SpO_2_ and the rise in CO_2_ (PtCO_2_, ETCO_2_, and PaCO_2_) with no major changes in the heart rate in our meta-analysis also transpires to be an unexpected reaction.

Sukul et al. (26) reported altered breathing patterns, respiratory resistance and discomfort under medical masks. Adults younger than 60 years of age described slow breathing (slow and deep inspiration and expiration) under masks, whereas shallow/thoracic breathing (breathing with increased inhalation duration and effort), respiratory resistance and dyspnea was portrayed by those ≥ 60 years of age. Fittingly, altered breathing patterns/kinetics, progressive changes toward deoxygenation, hypercarbia and insignificant changes in the respiratory and heart rate transpired to be surprising mask outcomes in our present results (hypercapnia-like effects). Thus, prolonged masks use may lead to hypercapnic hypoxia like conditions. While short and acute hypercapnic hypoxia like conditions in healthy individuals can promote positive effects (sport, training, etc.) (143–145), a chronic/prolonged hypercapnic hypoxia (as also known from sleep apnea) is toxic for the renal (146), nervous (147), and cardiovascular system (148) in the long run—causing metabolic syndrome (14) as well as additional effects on cognitive functions (149).

### N95 mask compared to surgical mask

In line with recent findings by Kisielinski et al. (14) and Sukul et al. (26), the present results clearly show that N95 masks lead to significantly more pronounced and unfavorable biochemical, physiological and psychological effects (Figure 7) than surgical masks. Altogether, the results in blood oxygenation, discomfort, heart rate, CO_2_, exertion, humidity, blood pressure, V_E_, temperature, dyspnea, and itching etc. can be attributed to the larger (almost doubled) dead space and higher breathing resistance of the N95 mask (14). Compared to the surgical mask upon the short-term effects, N95 masks could impose elevated health risks under extended use. Interestingly, recent data from a large multi-country RCT study show no significant differences between the two mask types in terms of SARS-CoV-2 infection rates (150). Nevertheless, there was long enforcement of N95 masks in e.g., Austria and Germany (9).

The article "Physio-metabolic and clinical consequences of wearing face masks—Systematic review with meta-analysis and comprehensive evaluation" was retracted in 2023. Reasons: concerns about the data; concerns about the results or conclusions.

### Short mask experiment times

It is noteworthy to say that in studies with short assessment times neither correspond to real-life conditions nor do they exclude short- or long-term compensatory mechanisms, e.g., obvious for CO_2_-rebreathing. Short mask experiments are also unable to show long-term changes. However, immediate compensatory mechanisms can hide further adverse reactions (122, 138, 140). Therefore, longer observation times can lead to clearer values that are closer or above the thresholds due to the attenuation or collapse of transient physiological mechanisms. The experimental studies used here examined important outcomes only had a median examination time of 18 min (Figure 11). Heterogeneous studies with small sample sizes yielded significant and medium to strong results (Figures 10, 12). Nevertheless, experimental studies with longer assessment periods are needed.

**Figure 11:** Illustration of the duration of studies in which measurements were made on mask effects (physical, biochemical, and physiological) in 934 participants. The median is 18 min (yellow dotted line) with an interquartile range of 50. The study with the longest experimental duration included 21 subjects, corresponding to 2.2% of the total population studied. Striking not only is a very short trial time compared to the everyday scenarios workday and school attendance (see interrupted, auxiliary lines in blue and red), but also a strongly deviating mask exposure duration with outliers (mean of 45.8 min with standard deviation of 69.9). Therefore, the mean is not an appropriate parameter to characterize this distribution.

**Figure 12:** Summary of pooled meta-analytic evaluation of face mask-wearing sensations measured with standardized Borg-. Likert-, VAS-scales, or similar. The height of the bars reflects the SMD (standard mean difference), their error bars correspond to the confidence intervals. Five out of 6 complaint categories (83%) are above the strong effect size threshold of >0.8 of the standard mean difference values according to Cohen (102). The meta-analytical statistical data were as follows (SMD = standard mean difference): Itch: SMD +1.57, 95 %CI −0.08 to 3.23, *Z* = 1.86, *p* = 0.06; Shortness of breath: SMD +1.46, 95% CI 0.42 to 2.50, *Z* = 2.75, *p* = 0.006; Discomfort: SMD +1.16, 95% CI 0.58 to 1.73, *Z* = 3.94, *p* < 0.0001; Exertion: SMD +0.9, 95% CI 0.57 to 1.23, *Z* = 5.31, *p* < 0.00001; Humidity: SMD +0.9, 95% CI 0.34 to 1.46, *Z* = 3.17, *p* = 0.002; Heat: SMD +0.77, 95% CI 0.29 to 1.26, *Z* = 3.11, *p* = 0.002.

The article "Physio-metabolic and clinical consequences of wearing face masks—Systematic review with meta-analysis and comprehensive evaluation" was retracted in 2023. Reasons: concerns about the data; concerns about the results or conclusions.

The observational studies included in the present analysis on symptoms were conducted over significantly longer periods (median 240 min, IQR 180) and are able to consider cumulative and long-term effects. It is known that observational studies are far more precise in finding negative effects and are particularly suitable to investigate exposures (e.g., air pollution or smoking) that are difficult or impossible to investigate in randomized controlled trials (RCTs). In addition, observational studies are important to investigate causes with a long latency period, such as toxicological and carcinogenic effects from environmental exposures or drugs (49).

The longest period of included studies was 8 months with an averaged of wearing the mask 8 h per day (observational study), however with the shortest study with a 5 min examining/exposition time (controlled trial).

### Possible sub-threshold impact of masks—The low-dose long-term effect on health

In contrast to our study, most of the recent systematic reviews (27–31) have only analyzed a few outcome threshold values without considering comprehensive effects, exposure time and the susceptibility of the exposed organisms and tissues. Therefore, their recommendations e.g., masks are harmless and safe for everybody etc. appears to be superficial, non-medical, non-holistic, and misleading.

In accordance with conclusions of Sukul et al., Fikenzer et al., and Zhang et al. (26, 53, 62), we have found hints to deleterious effects even without exceeding physiological threshold values and we have interpreted these data as a risk for individuals with suppressed compensatory mechanisms such as in older individuals and sick subjects with cardiorespiratory diseases, infection, diabetes, cancer, and other comorbidities. Sukul et al. (26) were able to show that the unfavorable effects are more pronounced in the older adults (aged: 60–80 years). Moreover, they could provide evidence for toxic effects of face masks including oxidative stress, immunosuppression, deoxygenation and hypercarbia induced vasoconstriction and altered systemic microbial activity.

The article "Physio-metabolic and clinical consequences of wearing face masks—Systematic review with meta-analysis and comprehensive evaluation" was retracted in 2023. Reasons: concerns about the data; concerns about the results or conclusions.

Even with CO_2_ and SpO_2_ levels that do not exceed the limits, many clinical researchers have also found troubling results in face mask wearers.

Neurologists observed changes in MRI brain signal baseline level due to face mask use (15). Wearing a surgical mask for merely 9 min increased end-tidal CO_2_ causing mild hypercapnia. This was responsible for a compensatory increase in cerebral blood flow with morphological changes similar to that of a CO_2_ gas challenge or holding your breath. In patients with aneurysms or brain tumors this phenomenon could be deleterious. Another study showed a pathologic and altered brain metabolism while wearing a N95 mask for 6 h (17). The MRI imaging revealed a significant drop in brain oxygenation. A more than 50% drop in oxygenation in the cingulate gyrus (cognition circuit) after 6 h of mask use was associated with clinical symptoms of a confused state in 80% of the subjects above 35 years. The authors even concluded that the general population should not wear a N95 mask. This phenomenon of brain deoxygenation could be dangerous for people with altered brain functions when on medication, after a transient ischemic attack (TIA) or stroke, respectively.

Ophthalmological studies indicated risk of retinal damage from long-term use of masks. N95 masks reduced the vascular density in the vascular plexus even under resting conditions as early as after 60 min (151). Here, the drop in SpO_2_ and increase in blood pressure were significant but within the normal physiological range. Another study reported a significant mask-induced increase in intraocular pressure (IOP) after ~5 min of wearing (12). Thus, wearing masks may counteract the therapy aiming to reduce the IOP and can exacerbate irreversible long-term vision problems in individuals with glaucoma. Numerous other studies have shown that the long-term effects, leading to deleterious clinical outcome may result from prolonged mask wearing (15, 17, 151, 152). Such effects are comparable to sick building syndrome (SBS) (153), cigarette smoking and other chronic, slightly toxic influences relevant to the general population.

In accordance with our present analysis and precedent scoping review (14), mask-related changes in leaning toward pathological values can lead to illness and clinical consequences, just like chronically, repeated subliminal harmful environmental events. Occupational diseases defined by the International Labor Organization (ILO) and that are in accordance with the worker's compensation act in Germany illustrates the potential harm caused by chronic exposure to subthreshold environmental factors (154). Numerous examples of these principles can be found in the literature concerning pharmacology, toxicology, clinical and occupational medicine and even in psychology (155–164). Many other toxicological and environmental health examples are presented in the recent scoping review by Kisielinski et al. (14), which refers to MIES (Mask-Induced Exhaustion Syndrome). Such subliminal chronical changes and harmful effects in the long run are comparable to the sick building syndrome (SBS) (153), cigarette smoking (165), salty diet (166), aluminum environmental pollution (167), low-level lead exposure (168), organochlorine pesticides and polychlorinated biphenyl exposure (169), or even the so-called climate change exposure (170).

The article "Physio-metabolic and clinical consequences of wearing face masks—Systematic review with meta-analysis and comprehensive evaluation" was retracted in 2023. Reasons: concerns about the data; concerns about the results or conclusions.

Altogether, even the subliminal changes due to face mask use can become clinically relevant.

### Overlapping of face mask effects (MIES) with long-COVID-19 symptoms

Regarding the numerous mask symptoms an important question arises: Can masks be responsible for a misinterpreted long-COVID-19-syndrome after an effectively treated COVID-19 infection? Nearly 40% of main long-COVID-19 symptoms (171) overlap with mask related complaints and symptoms described by Kisielinski et al. as MIES (14) like fatigue, dyspnea, confusion, anxiety, depression, tachycardia, dizziness, and headache, which we also detected in the qualitative and quantitative analysis of face mask effects in our systematic review. It is possible that some symptoms attributed to long-COVID-19 are predominantly mask-related. Further research on this phenomenon needs to be conducted.

### Complaints and symptoms under mask use and the WHO definition of health

Amongst the perceived sensations with mask use only six symptoms (exertion, discomfort, shortness of breath, humidity, heat, and itch) could be meta-analyzed and have resulted in predominantly strong effect sizes (Figure 12). In the pooled prevalence analysis, we included eight main symptoms namely headache, acne, skin irritation, shortness of breath, heat, itch, voice disorder, and dizziness (Figure 13) out of which all were significant in the evaluated population (Figure 8). There are many more reported in the literature. However, these could not be meta-analyzed due to the low number of comparable studies on those particular complaints. In the included literature additional reported mask related symptoms were: rhinitis (80), difficulties to think and to concentrate (81, 94, 95, 101), drowsiness (95), communication disorder (88, 94, 99), depression and mood swings (75, 76, 88, 92), anger (92), perceived discomfort (47, 52, 53, 69), anxiety (75, 88, 92), and an overall perceived fatigue and exhaustion (52–54, 57–62, 68, 70, 71, 73, 79, 83, 94).

The article "Physio-metabolic and clinical consequences of wearing face masks—Systematic review with meta-analysis and comprehensive evaluation" was retracted in 2023. Reasons: concerns about the data; concerns about the results or conclusions.

**Figure 13:** Representation of symptom prevalence in % during face mask use as the area of the circles. Along the X-axis, the main recorded symptoms are listed. The higher the prevalence, the bigger the circles and the more often the symptoms. The Y-axis gives the probability of non-random occurrence of the symptoms and includes the statistical Z-value. Thus, the higher the circles are arranged, the more robust is the relationship to face mask wearing. The meta-analytical statistical data were as follows: Headache: 62% (95% CI 48–75%), *Z* = 8.77, *p* < 0.00001; Acne: 38% (95% CI 22–54%), *Z* = 4.58, *p* < 0.00001: Skin irritation: 36% (95% CI 24–49%), *Z* = 5.61, *p* < 0.00001; Shortness of breath: 33% (95% CI 23–44%), *Z* = 6.28, *p* < 0.00001; Heat: 28% (95% CI 15–0.37%), *Z* = 4.72, *p* < 0.00001; Itch: 26% (95% CI 15–36%), *Z* = 4.77, *p* < 0.00001; Voice disorder 23% (95% CI 2–43%), *Z* = 2.15, *p* < 0.03; Dizziness 5% (95% CI 1–9%), *Z* = 2.5, *p* = 0.01.

All of these mask-related symptoms contradict a state of wellbeing and health as defined by the WHO. According to the WHO; “health is a state of complete physical, mental, and social wellbeing and not merely the absence of disease or infirmity” (172). Based on our findings, the use of face mask in the hope of maintaining health is unfortunately contradicting the WHO's definition of health. Regarding all the possible side effects of mask and their still unproven efficacy against viral transmission within the general population (5, 10, 173, 174), health seems not to be substantially preserved by wearing face masks. So far, only two randomized controlled mask trials for prevention of SARS-CoV-2 infection in the general population have been published: one high quality study from Denmark, Europe (175), and the other from Bangladesh with biased results and a lot of inconsistencies (176). Based on a Bayesian random-effects meta-analysis of these two trials, the posterior median for relative risk was 0.91 (95% credible interval 0.63–1.33, 73% probability of some benefits with very limited evidence) (177). Recent data from a large multi-country RCT study show no significant differences between the surgical and N95 mask in terms of SARS-CoV-2 infection rates (150). Asides, there is evidence that COVID-19 rates have been able to expand swiftly when omicron hit (178) even in societies where mask use was assiduously followed—as in Korea, Taiwan, Hong Kong, and Singapore (179). The paucity in high-quality mask studies is unfortunate. Seeing the overall weak evidence for efficacy of masks against viral transmission within the general population (5, 10, 173, 174, 180–184), face masks have to be evaluated appropriately in the sense of the *Hippocratic Oath* and as per the *Primum nihil nocere* (above all do not harm). To avoid at all costs that the damage caused by preventive or therapeutic measures becomes greater than that caused by the disease itself, should be the credo of all those involved in the containment of the crisis, including politicians and the so-called experts. Medical decisions can only be made on the basis of comprehensive knowledge on a patient's overall condition, individualized case history, considering all previous illnesses and interventions, physical and mental predispositions, and his/her socio-economic state, etc. When it comes to medical decision-making in a sick person, the weighing of therapeutic measures for the benefit of the patient against the side effects of the therapy is to be evaluated differently than a prophylactic procedure in healthy people. If wrong decisions are made in the selection of preventive measures in healthy individuals, or if they are improperly applied, the consequences are usually much more severe and liability claims are often unavoidable. From a standardization point of view the filtration efficacy of mask for viruses remains hypothetic and not in line with the established standards. There are national and international standards for bacteria filtration efficiency (BFE) for medical masks since decades, for example the EU-EN 14683, or the USA-ASTM F2101. They are the prerequisites for general approval. However, since 2020 (i.e., nearly 3 years), no comparable standard/testing of masks for viruses does yet exist. Given the fact, that medical masks (surgical and N95) increase particle exhalation in the smallest size range of 0.3–0.5 μm, shifting the geometric mean diameter toward smaller sizes (longer in air) compared to no mask conditions (185) doubts arise. Such scientific facts are pointing toward the nebulization effect of masks, which could be an add-on for their weakness against viral transmission in general.

The article "Physio-metabolic and clinical consequences of wearing face masks—Systematic review with meta-analysis and comprehensive evaluation" was retracted in 2023. Reasons: concerns about the data; concerns about the results or conclusions.

## Limitations

Our systematic review rarely discussed the inhaled toxins associated with the mask. Inhalation and ingestion of toxic substances, which are ingredients of the masks, are also of importance in evaluating this pandemic non-pharmaceutical intervention (NPI). In addition, our work has not extensively studied the microbial colonization of masks and the consequences of contamination by microorganisms for the wearer.

In our meta-analysis ETCO_2_ and PtCO_2_ have been used as an approximation of PaCO_2_ (44–46). Therefore, the real PaCO_2_ values could be slightly higher or lower. The median exposure period for most studies evaluating physio-metabolic mask adverse effects was 18 min. There are few experimental studies evaluating mask adverse effects for longer periods that would more closely reflect real-world use. Therefore, the negative physio-metabolic and clinical effects of the face masks may well be worse than we have determined.

Based on the studies conducted during the pandemic, the control groups without masks were mostly the same individuals, or individuals who were not mask abstinent for too long (general mask requirement) (186), so the mask-no-mask differences may be mitigated.

Because of the rapid flow of science, new relevant papers have certainly appeared that we were unable to consider in the meta-analysis as they appeared after the period of our data search (search limitation to 31.12.2021). The most important and relevant observational studies were considered for this analysis thereby addressing the physio-metabolic and clinical effects.

Numerous psychological and social effects could not be assessed analytically as too few relevant and evaluable studies were available. However, the simplest and clearest face mask harms, over and above the physiological and clinical discussed here, are the psychological and social ones—impeding communication visually and verbally (187–189), disturbed facial expressions and misinterpretation of emotions (190), with the consequence of impeded early childhood learning (191).

## Conclusion

This systematic review comprehensively revealed ample evidence for multiple adverse physio-metabolic and clinical outcomes of medical face masks, with worse outcomes in the case of N95 masks. This can have long-term clinical consequences, especially for vulnerable groups e.g., children, pregnant, older adult, and the ill. Besides transient and progressive hypoxemia, hypercarbia, and individualized clinical symptoms our findings are in line with reports on face masks caused down-stream aberrations (e.g., oxidative stress, hypercapnia, vasoconstriction, pro-inflammatory response, immunosuppression etc.) at the organ, cellular and microbiome levels and support the MIES (Mask Induced Exhaustion Syndrome). From our point of view, while a short application of the mask seems to be less harmful, longer and long-term use may cause shift toward the pathophysiological direction with clinical consequences even without exceeding physiological thresholds (O_2_ and CO_2_).

So far, several MIES symptoms may have been misinterpreted as long COVID-19 symptoms.

In any case, the possible MIES triggered by masks contrasts with the WHO definition of health.

The exact threshold of harmless and non-pathogenic time wearing a mask should exclusively be determined by further intensive research and studies. Due to the ultimate lack of exclusion of the harmfulness of mask wearing, mask use by the general public should be discouraged.

The article "Physio-metabolic and clinical consequences of wearing face masks—Systematic review with meta-analysis and comprehensive evaluation" was retracted in 2023. Reasons: concerns about the data; concerns about the results or conclusions.

In the sense of effectiveness of face masks in the real-world setting (cost-benefit), the mask should show a benefit in terms of reduced respiratory infections, e.g., in healthcare through fewer consultations or hospitalizations (192). Unfortunately, this was not the case, e.g., in Germany (193) and USA (194), where mask mandates were ubiquitous (9). Additionally, there is evidence that COVID-19 rates have been able to expand swiftly when omicron hit (178) even in societies where mask use was assiduously followed—as in Korea, Taiwan, Hong Kong, and Singapore (179).

From the above facts, we conclude that a mask requirement must be reconsidered in a strictly scientific way without any political interference as well as from a humanitarian and ethical point of view. There is an urgent need to balance adverse mask effects with their anticipated efficacy against viral transmission. In the absence of strong empirical evidence of mask effectiveness, mask wearing should not be mandated let alone enforced by law.

## Data availability statement

The original contributions presented in the study are included in the article/supplementary material, further inquiries can be directed to the corresponding authors.

## Author contributions

KK, AS, and OH: conceptualization and methodology. KK and OH: software. KK, OH, SW, BW, SF, AP, BK, SK, PS, and AS: formal analysis and writing—review and editing. KK, OH, SW, BW, PS, and AS: investigation. KK, SW, SF, BK, AP, PS, and AS: physio-metabolic and clinical interpretations. KK, OH, PS, and AS: writing—original draft preparation. All authors have read and agreed to the published version of the manuscript.
